# Machine Learning and Electrocardiography Signal-Based Minimum Calculation Time Detection for Blood Pressure Detection

**DOI:** 10.1155/2022/5714454

**Published:** 2022-07-19

**Authors:** Majid Nour, Derya Kandaz, Muhammed Kursad Ucar, Kemal Polat, Adi Alhudhaif

**Affiliations:** ^1^Department of Electrical and Computer Engineering, Faculty of Engineering, King Abdulaziz University, Jeddah 21589, Saudi Arabia; ^2^Electrical-Electronics Engineering, Faculty of Engineering, Sakarya University, 54187 Sakarya, Turkey; ^3^Department of Electrical and Electronics Engineering, Faculty of Engineering, Bolu Abant Izzet Baysal University, Bolu 14280, Turkey; ^4^Department of Computer Science, College of Computer Engineering and Sciences in Al-Kharj, Prince Sattam Bin Abdulaziz University, P.O. Box 151, Al-Kharj 11942, Saudi Arabia

## Abstract

**Objective:**

Measurement and monitoring of blood pressure are of great importance for preventing diseases such as cardiovascular and stroke caused by hypertension. Therefore, there is a need for advanced artificial intelligence-based systolic and diastolic blood pressure systems with a new technological infrastructure with a noninvasive process. The study is aimed at determining the minimum ECG time required for calculating systolic and diastolic blood pressure based on the Electrocardiography (ECG) signal. *Methodology*. The study includes ECG recordings of five individuals taken from the IEEE database, measured during daily activity. For the study, each signal was divided into epochs of 2-4-6-8-10-12-14-16-18-20 seconds. Twenty-five features were extracted from each epoched signal. The dimension of the dataset was reduced by using Spearman's feature selection algorithm. Analysis based on metrics was carried out by applying machine learning algorithms to the obtained dataset. Gaussian process regression exponential (GPR) machine learning algorithm was preferred because it is easy to integrate into embedded systems.

**Results:**

The MAPE estimation performance values for diastolic and systolic blood pressure values for 16-second epochs were 2.44 mmHg and 1.92 mmHg, respectively.

**Conclusion:**

According to the study results, it is evaluated that systolic and diastolic blood pressure values can be calculated with a high-performance ratio with 16-second ECG signals.

## 1. Introduction

### 1.1. Background and Motivation

The state of blood pressure higher than usual is called hypertension [1]. Hypertension is a risk factor for many cardiovascular diseases such as stroke, renal failure, and heart attack that affect many people today [2–4]. Hypertension is responsible for one out of every two deaths in the world [3]. However, with BP data from 1.7 million people in 31 provinces of China, many people with or without hypertension or advanced disease have been identified, and they have developed methodologies for awareness, diagnosis, and control of the disease [5]. The level of importance is emphasized in the study conducted in a country with a significant population such as China. However, continuous blood pressure monitoring is essential for diagnosis and treatment.

BP monitoring is an essential factor in the early diagnosis and treatment of hypertension [2, 3]. When the heart muscle contracts, systolic blood pressure occurs, and diastolic blood pressure occurs when it relaxes. In other words, high BP is an indicator of the pressure exerted by the blood on the blood vessels [1, 3, 6]. SBP is about 80 mmHg, and DBP is about 120 mmHg. Hypertension is defined as above 140 mmHg SBP and 90 mmHg DBP. If the BP is above average, the heart starts to work harder. An imbalanced heart causes swelling in the vessels, blindness, and heart failure causes many diseases [3]. Since the heart meets the nutritional needs of all organs, imbalances in the heart indirectly affect other organs. In this case, hypertension affects many organs, especially the brain and kidneys [1–3].

Although the gold standard is mercury methods in BP monitoring, many methods have been developed today [3, 7]. Due to the toxic effects of mercury, reliable electronic devices are recommended by the World Health Organization [3].

According to the World Health Organization, the hypertension diagnosis algorithm is as follows [3]. (1) A few days of registration should be taken. (2) Measurements should be made twice a day, in the morning and the evening. (3) Two consecutive measurements are taken with at least one minute between them in each measurement. The average value of the measurements is taken. (4) Measurements are taken in the sitting position. Although a few daily measurements are considered sufficient by the World Health Organization, a one-week follow-up is recommended in some studies [8].

Studies show that drug treatments can control hypertension [1, 9]. In patients with hypertension, the disease and drug treatment follow-up are vital. For this reason, it is recommended that patients follow their treatments meticulously [1, 3, 9].

In the past, BP measurements were made in health centers since devices for BP measurements were not widely used. However, today, with the widespread use of BP measuring devices, the possibilities of measuring at home have increased. The most important feature of the devices was that individuals could measure without the need for technical knowledge [7, 10]. Although the devices are easy to use, measurement accuracy is vital. For this reason, it is recommended to prefer verified devices [10].

Each device can use a different measurement technique and location [7]. However, the World Health Organization recommends measurement from the upper arm in a sitting position [3]. It is known that upper arm measurement produces more accurate results than wrist measurement [3]. In patients who cannot be in every position, such as pregnant, there is a significant change in the results because the measurement standard is exceeded [11].

Although BP monitors take measurements from different places and calculate BP with different methods, they are subject to the same design protocols. There are many protocols in the literature [10]. The aim of all of them is to develop a quality measuring system. The International Organization for Standardization (ISO) [12], the European Society of Hypertension International Protocol (ESH-IP) [13–15], and the Association for the Advancement of Medical Instrumentation (AAMI) standard [16] are just a few of them.

Noninvasive brachial BP measurement is a primary method in diagnosing hypertension diseases [17, 18]. However, this measurement creates significant problems for public health. Every year, in American states, it has been determined that the BP measurement of approximately one million people is measured above or below normal by 5 mmHg. With the resulting extra costs, people have suffered the adverse effects of the wrong treatment [17]. For this reason, it is essential to determine the correct BP measurement method. There are many BP estimation methods in the literature, such as auscultatory methods, plethysmography, tonometry, and oscillometric methods [7, 10]. Although cuffed devices have been produced for many years, the new target is to measure BP without causing discomfort to the patient [10, 19]. Noninvasive methods, including PPG- and electrocardiography- (ECG-) based signal processing and artificial intelligence, are promising BP measurement methods [10, 19, 20].

Many methods with invasive and noninvasive structures are used in BP measurements. Invasive measurement systems often cause problems such as incorrect measurements and loss of time. However, noninvasive models cause many problems, such as ease of use and hardware and software costs. If it is mentioned in a few articles in the literature that these problems are seen, the initial states of the model designed with a neural network using a genetic algorithm were tried to be optimized, but this caused problems in terms of time and hardware cost and caused only a tiny change in the accuracy rate. While the impact of BP measurements on human life is of such high importance, developing these systems is of great importance for researchers. For BP measurement models, each study applies a different methodology. This study takes its place with a different approach between these studies, which differ in their superiority to each other. A study on the determination of blood pressure measurement time has not been found so far. For this reason, the study presents an original model. Instead of complex and sophisticated mathematical expressions seen in deep learning algorithms, a model based on machine learning techniques has been developed. In addition, the findings obtained in the literature review show that the designed model has a higher accuracy rate than other models.

Signal processing, spectrum segmentation, feature extraction applications, and morphological filters are used in many fields. In this study, signal segmentation and feature selection were performed. These processes occur not only in fields such as biomedicine, medicine, and image processing but also in engineering and commerce. It has applications with various methodologies in different fields. Tabatabaei et al. performed signal analysis with acoustic emission method (AEM) to detect defects on angular contact bearings. The authors applied feature extraction with empirical mode decomposition (EMD) algorithm on the signals obtained with AEM [21]. EMD is used to analyze nonlinear and nonstationary signals by separating them into components with different resolutions [22]. Using this method, the authors extracted intrinsic mode functions from the signals as if they were extracting time and frequency domain properties, and by transforming these functions into an analytical expression with Hilbert transform, they created a model that can detect defects on bearings. However, the same application process has been applied by different authors in classifying electroencephalography (EEG) signals as seizure and nonseizure [23]. EEG signals are decomposed into intrinsic mode functions by the EMD method. These functions were converted into an analytical expression and extracted from the bandwidth properties of the signals. Classification based on ML techniques was created at the end of the model. Two articles with similar content applied the exact solution to different problems. In yet another article, different domain properties were used to detect defects on angular contact bearings, which is one of the crucial subgroups of bearings, and as a result, the model that would make the best defect detection was realized by using time-domain properties [24]. Zhang and Wang extracted 21-time domain features for BP detection from PPG signals [25]. They provided the size optimization with mean impact value (MIV). By calculating the effect factor on the signals of each feature, they extracted 8 features with a shallow impact. He created a new model by optimizing the initial conditions of the neural network, the last used ML technique, with the genetic algorithm. This article, which has the same research subject, has created its model with a specific approach [25]. However, considering that the amount of features used is high, the use of optimization algorithms causes a minimal change in the accuracy of blood pressure detection, and it is thought that it will be expensive in terms of hardware cost. It is concluded that it is not a good model.

The development of machine learning algorithms makes it possible to create innovative models for the same problem. The article's methodology is presented step by step by addressing such processes. First, signal processing is applied so that the signals can be used efficiently. There are many studies based on signal processing in the literature. These are frequently preferred because they are noninvasive methods [26–28]. Although its measurement is relatively difficult compared to PPG, some studies use oscillometric waveforms [29, 30], auscultatory and oscillometric waveforms [31], and peripheral signals [26]. In addition to these, speech-based measurement methods are also available [32]. These studies applied signal processing processes, and machine learning algorithms were used in BP estimation according to the need. PPG and ECG are a group of biomedical signals that are very easy to measure. ECG can be easily measured on bedside monitors and Holter devices. On the other hand, PPG can now be measured even on intelligent wristbands. For this reason, interest in ECG- and PPG-based BP estimation studies has increased in the literature [10, 19, 20]. ECG signals were preferred in this study because they are easy to measure.

Signal processing studies include digital filtering, feature extraction, feature selection, and machine learning-based regression steps [20, 27, 33]. In the case of using deep learning, feature extraction and selection operations are performed by deep learning [34]. The success of the signal processing process depends on the designed steps. The feature extraction steps often focuses on the formal properties of the signals [29–31]. In the event of deformities, the system's collapse is expected. However, examining the statistical properties of the signal instead of the formal properties will reduce the errors and help catch the overlooked information [35–37]. In this study, 25 statistical-based features were extracted instead of the standard features used in the literature.

Although deep learning methods include feature extraction and selection steps, the training periods are pretty long [20, 28, 34]. Compared to classical machine learning algorithms, the success rate of deep learning is relatively high. This study proposes a method based on classical machine learning algorithms by optimizing signal processing processes. This study's Gaussian process regression (GPR), regression tree ensembles, and regression trees were preferred because of their high-performance [38–40].

Feature selection algorithms are generally not preferred in BP estimation studies [26, 27, 31]. In studies where classical machine learning algorithms are preferred, model performance is increased using feature selection algorithms [41–43]. The Spearman correlation coefficient-based feature selection algorithm was preferred in this study due to its high performance.

In the literature, studies on BP estimation seem to be one step ahead of learning-based studies [20, 28, 32]. Model performance values in BP estimation models developed with ECG and PPG signals are 0.84 < *R* < 0.95, 3.36 < MAE < 5.48, and 0.78 < RMSE < 13.83 [20, 33, 34]. In a study with auscultatory and oscillometric waveforms, the model performance was −0.9 < MAE < 11,032 and 0.423 < *R* < 0.948.

Although models have been developed in the literature, there is no information about how many seconds the models can measure. This study is aimed at determining the minimum duration of ECG signal required to estimate SBP and DBP with ECG. Firstly, ten different datasets were created in the study by dividing the ECG signal into epochs of 2, 4, 6, 8, 10, 12, 14, 16, 18, and 20 seconds. Then, 25 features were extracted from each epoch in the time domain. With the help of the Spearman feature selection algorithm, relevant features were selected, and BP values were estimated with the help of machine learning algorithms.

### 1.2. Literature Review

Machine learning, the application of artificial intelligence, creates a paradigm shift in medicine with its features in pathological diagnosis, patient monitoring, and helping treatment [44]. Numerous studies are being conducted on the relationship between biomedical signals and blood pressure for the appropriate and timely treatment of hypertension using machine learning algorithms [45]. A typical biomedical signal processing system includes the biological system of interest, the sensors used to capture the activity of the biomedical system, and the process of extracting the appropriate methodology to analyze the signals and extract the desired information from the relevant signal. The biological signal examined in this study is the ECG signal, which shows the heart's electrical activities.

Recent technological advances have made wearable biosensors suitable for daily use. Wearable biosensors provide an opportunity for real-time monitoring of vital human signs, providing timely feedback, and providing early diagnosis and treatment possibilities [46, 47]. Unlike conventional BP sensors, which are subject to a specific measurement procedure, modern wearable biosensors monitor the relevant signals all day long and do not create a burden other than wearing the device. Reliably receiving these signals from the human body and collecting the received signal data brings along important research [48–50]. Securely collecting, verifying, and transporting electronic data is achieved through the integration of the internet of things (IoT) and artificial intelligence technology [51–53]. The difficulty of effectively guaranteeing the quality of IoT equipment brings with it the difficulty of ensuring the reliability and accuracy of the data [54, 55]. This situation is of great importance in the accuracy of algorithms based on ML techniques. Ahamed and Farid states that datasets produced with IoT terminals cannot fully cover medical scenarios, and intelligent diagnosis will be significantly reduced [56]. However, advances are currently being made in IoT, allowing high-reliability acquisition of medical image data and multiwaveform data [57]. Good results are obtained from such devices in real-life conditions. Superficial temporal artery tonometry-based device [58], PPG optical sensor [59], ARTSENS (Arterial Stiffness Assessment for Noninvasive Scanning) pressure for brachial arterial pressure [60], a BP estimator based on the principle of volume compensation citeTanaka2007, and the Modulated Magnetic Blood Signature mechanism [61] noninvasive are some of the measurement systems developed for BP monitoring.

Most research on blood pressure estimation uses either electrocardiogram and photoplethysmograph signals or a combination. While this causes more problems, it also brings with it the need for equipment. Taking PPG signal measurements requires the use of many techniques [62–65]. Proper use of these techniques requires accurate measurement of PPG signals. Therefore, the use of PPG signals for BP measurement is not a correct option [66, 67]. This study, on the other hand, is aimed at estimating BP with the dataset created by extracting statistical features from ECG signals.

### 1.3. Aims and Contributions

In real-life situations, in vehicles, at home, or in hospitals, BP can only be measured with a stand-alone BP device. On the other hand, modern telemedicine allows the development of biosensors in electrodes attached to the patient's chest, allowing the measurement of BP to be obtained. The proposed method offers usage areas ranging from clinical situations to military environments with wearable sensor technology. In addition, a suitable methodology has been developed to reduce the need to connect various sensors to the human body. The developed model is aimed at determining the SBP and DBP estimation time based on artificial intelligence-based ECG signals. Although there are many studies in the literature that detect blood pressure with ECG, there has been no study on how long blood pressure can be measured.

## 2. Methodology

The basic approach to providing BP estimation is shown as a flow diagram in Figure 1. The process given in the flow chart was applied step by step. First, the ECG signals are sourced from the IEEE open-source data-sharing platform [68, 69]. In the received dataset, epoching was applied to estimate BP in the shortest possible time frame for ECG signals. After this step, the time domain features of each ECG signal are taken for feature extraction. Derived features are used as inputs for various machine learning algorithms. Finally, a suitable feature selection algorithm was applied to the model to increase the performance. The described process will be discussed in detail in the following sections.

### 2.1. Data Preprocessing

#### 2.1.1. Data Acquisition

In this study, the open-source dataset on the IEEE database sharing platform was used [68, 69]. In this dataset, there are ECG, PPG, and BP records. These records were obtained from five young, healthy individuals (one female and four male) who did not have peripheral or cardiovascular disease and ranged from sedentary to regular activity levels. The dataset was created by taking records for six and a half hours each day for three days. Example ECG signals of these individuals are given in Figure 2.

#### 2.1.2. Epoching

The ECG signal with a sampling frequency of 64 Hz was split into epochs of 2-4-6-8-10-12-14-16-18-20 seconds to generate the BP prediction model. SBP and DBP signals were obtained for each period. Example ECG and BP signals of the 4-second epoch are given in Figure 3.

Figure 3 contains simultaneous BP signal for 4-second ECG recording. The BP signal has four maximum and minimum points for 4 seconds. The minimum points of the BP signal represent DBP, while the maximum points represent SBP. DBP and SBP values are calculated over these points. SBP corresponds to the average of the maximum points and DBP to the average of the minimum points. If Figure 3 is examined in detail, it will be observed that there are similar characteristics of ECG and BP signals.

### 2.2. Feature Extraction

The five simultaneous ECG signals obtained must have certain inputs for the machine learning algorithms to be applied. These inputs are descriptive parameters often used in statistical science. Descriptive parameters include information such as standard deviation, central moment, IQR, and 25 in total. A total of 125 features were extracted from five signals (Table 1). Here, feature extraction is aimed at obtaining ECG signal information with the help of different parameters by preventing information loss.

### 2.3. Feature Selection Algorithm

In other words, feature selection, called size optimization, is an algorithm that eliminates irrelevant features in the dataset [32]. Feature selection is applied to increase the performance of machine learning algorithms and reduce the size of the dataset containing the feature entries and the computational load [27]. Many parameters are used to calculate the level of relationship between features in statistics. This study used a Spearman correlation coefficient-based feature selection algorithm for feature selection.

#### 2.3.1. Spearman Correlation Coefficients

Spearman's correlation coefficient (*r*_*s*_) is a statistical method used to express the level of correlation of features in a dataset with the label (SBP or DBP). It takes values between -1 and +1 [70]. While +1 indicates a perfect fit between the data, -1 indicates a negative perfect fit. 0 indicates that there is no relationship level. Accordingly, the level of relationship between SBP and DBP values and 125 features is presented in Table 2.

### 2.4. Machine Learning Algorithms

The study's machine learning algorithms are ensemble bagged tree, fine tree, and Gaussian process regression. These models have good performance, simple structure, and widespread use in regression problems [43]. The top three algorithms with the best performance were selected for use in a software environment with extensive machine learning algorithms. Performance monitoring of each epoched signal has been made for the selected ML techniques. The explanation based on the working principle of these algorithms is presented in detail in the following sections.

#### 2.4.1. Ensemble Bagged Tree: Prediction of SBP and DBP

Classification and regression trees (CART) is a machine learning technique developed by Breiman et al. (1984) [71]. The change in training sampling in the dataset causes an imbalance in the technique in question [72]. For this reason, the ensemble technique was preferred in the study. In addition, the nonlinear structure of the output values of the study data has been a good reason for the use of this method. It was created by combining several decision tree structures [73] to increase the performance value derived from a single decision tree structure. Ensemble has three methods: bagging, random forests, and boosting [72]. EBT was used to estimate SBP and DBP in the study. This model was designed based on a statistical method called boostrap [71, 74].

In bagging, many bootstrap samples are taken from the ECG signal training dataset. The regression model for each sample was carried out, the generated bootstrap samples were combined, and the model took its final form. The bagging predictor is determined by taking the average of this regression model. It is desired that the mean value is low, and the variance is high. For this reason, it is aimed that the algorithm structure that will perform the SBP and DBP estimation will work with a high accuracy rate. Accordingly, the performance of EBT on each epoched signal was determined.

#### 2.4.2. Fine Tree: Prediction of SBP and DBP

There are many original structures developed for CART [75, 76]. EBT, one of these structures, is explained in detail. The decision tree structure examined in the EBT is implemented using a single decision tree for this model. The model is designed by performing depth control with the split number of the decision tree. In addition, the decision tree is divided into fine, medium, and coarse according to the performance values (from best to worst) for certain split numbers in the software environment. A FT algorithm has been applied for the model design, which exhibits a reasonable prediction accuracy rate with its fit to the dataset.

Empirical evidence predicts that a correct, step-by-step decision tree is faster than a model in which the entire training dataset is tested and constructed. However, the final model of an iteratively designed tree cannot be reached without using the entire training set [77]. In addition to these contradictions, the model design must be clear, simple, and have a high accuracy rate. This study achieved the desired targets by keeping the number of splits to a minimum. SBP and DBP prediction models were created for each epoched signal. The highest performance ratio was obtained in the eleventh feature group. However, FT was observed to be low compared to the performances of other used EBT and GPR models. This can be explained as the dataset used does not fit well with the algorithm.

#### 2.4.3. Gaussian Process Regression: Prediction of SBP and DBP

Gaussian process regression (GPR), a Bayesian method, is a robust algorithm used for nonlinear regression models. Since the input parameters are nonlinear and more than one, SBP and DBP estimation were performed with this algorithm.

(1) $$\begin{array}{c} m\left(x\right)=E\left(f\left(x\right)\right),\;\forall_{x}\in X\left(\text{mean function}\right), \end{array}$$

(2) $$\begin{array}{c} k\left(x,x^{\prime }\right)=\text{Cov}\left(f\left(x\right),f\left(x^{\prime }\right)\right),\;\forall_{x},x^{\prime }\in X\left(\text{covariance function}\right). \end{array}$$

A Gaussian operation can be defined by its mean (1) and covariance function (2) [30]. The GPR covariance of the input variables is named as kernel or covariance function. The use of mean function and kernel function together refers to GPR.

### 2.5. Performance Evaluation Criteria

Mean absolute percentage error (MAPE-Equation (3)), mean absolute deviation (MAD-Equation (4)), standard error (SE-Equation (5)), mean squared error (MSE)-equation refMSE), root mean square error (RMSE-Equation (7)), *R*, and *R*^2^ are used in 7 parameters [43].

(3) $$\begin{array}{c} \text{MAPE}=\frac{1}{n}\overset{n}{\underset{i=1}{\sum }}\frac{\left|t_{i}-y_{i}\right|}{t_{i}}\times 100, \end{array}$$

(4) $$\begin{array}{c} \text{MAD}=\frac{1}{n}\overset{n}{\underset{i=1}{\sum }}\left|t_{i}-y_{i}\right|, \end{array}$$

(5) $$\begin{array}{c} \text{SH}=\sqrt{\frac{\sum_{i=1}^{n}{\left(t_{i}-y_{i}\right)}^{2}}{n-2}}=\sqrt{\frac{\sum_{i=1}^{n}{e_{i}}^{2}}{n-2}}, \end{array}$$

(6) $$\begin{array}{c} \text{MSE}=\frac{1}{n}\overset{n}{\underset{i=1}{\sum }}{e_{i}}^{2}, \end{array}$$

(7) $$\begin{array}{c} \text{RMSE}=\sqrt{\frac{1}{n}\overset{n}{\underset{i=1}{\sum }}{e_{i}}^{2}}. \end{array}$$

The dataset for training and testing is divided as specified in Table 3. The performance value of the model was evaluated for both split datasets.

## 3. Results

The study mainly aims to create models that can detect SBP and DBP estimation as soon as possible based on machine learning algorithms with ECG signals. In line with this goal, the application was carried out step by step according to the flow diagram given in Figure 1. First, the IEEE open-source data-sharing platform obtained a PPG, ECG, and BP information dataset. ECG and BP data from five individuals were used in the total. Afterward, the signals were epoched up to 20 at intervals of two seconds, starting from 2 for the epoching process. Since the dataset does not have input information, 25 feature extractions were made in the time domain. In order to achieve size optimization, feature selection was made in the next step. Performance evaluation based on the three best-performing machine learning algorithms was conducted for 11 selected feature sets. Finally, the algorithm that performs the estimation of SBP and DBP with the best performance ratio in the shortest time is expressed both graphically and numerically.

In the first part of the study, SBP models were prepared for each epochated signal (Tables 4–13). Twenty-five feature extractions were performed as ECG signal input information. Feature selection was carried out to reduce the size of the feature vector and get rid of the workload of unnecessary features. The correlation of 25 features was calculated by Spearman's method, and they were ranked from the highest correlation level to the lowest correlation level. Feature vectors were selected at 5% intervals according to the order. Initially, 5% of 25 features are taken (rounded to integers) to 1, 10% to 3, 15% to the fourth feature vector, up to 50%, 13. It was continued in the same way, and finally, the feature vector of the 25th column was obtained by taking 100%. Eleven groups were created with the ECG signal, and the performance evaluation table of 33 models was produced. According to this table, the best model is determined by dark color. EBT, the model created using all feature vectors (11 items), was the best performing algorithm with MAPE = 2.58 mmHg and *R* = 0.97 mmHg SBP values (Table 4).

The working process continued in the same way for the other epoched signals. For the 4-second epoch, SBP estimation models were created by evaluating the performance of each algorithm. A total of 11 groups were created with the ECG signal, and a performance evaluation table of 33 models was produced (Table 5). For the model constructed using all feature vectors, the EBT was the best performing algorithm with SBP values of MAPE = 2.34 mmHg and *R* = 0.97 mmHg. There are 25 feature vectors for the 6-second epoched ECG signal. The best-performing columns of these feature vectors were taken at 5% intervals, and performance evaluation was made for 11 features. For the 11th feature group, the best performing algorithm with MAPE = 2.27 mmHg and *R* = 0.97 mmHg SBP values were determined as EBT (Table 6). The same operations were performed for each epoched signal. The 11th feature vector per second was the best performing group. Accordingly, MAPE = 2.20 mmHg and *R* = 0.97 mmHg SBP values were determined for the 8-second epoch with the GPR algorithm (Table 7). According to the 10-second epoched ECG signal, MAPE = 2.08 mmHg and *R* = 0.97 mmHg SBP values were calculated using the EBT algorithm. Gradually improving performance values were calculated as MAPE = 2.04 mmHg and *R* = 0.98 mmHg for the 12-second epoched ECG signal (Table 8). Considering the increasing epoching times, the algorithm's best performance has varied each time. For the epoching times where the increase was observed, the GPR algorithm increased the *R* value while it caused a decrease in the MAPE value. For the 14-second epoch, SBP were obtained as MAPE = 2.00 mmHg and *R* = 0.98 mmHg (Table 10). For the 16-second epoch, SBP values were obtained as MAPE = 1.92 mmHg and *R* = 0.98 mmHg (Table 11). For the 18-second epoch, SBP values were obtained as MAPE = 1.97 mmHg and *R* = 0.98 mmHg (Table 12). For the 20-second epoch, SBP values were obtained as MAPE = 1.96 mmHg and *R* = 0.98 mmHg (Table 13).

While the *R* value did not change much before the 16th second, the MAPE value decreased. After the 16th second, the MAPE value decreases, while the *R* value decreases. MAPE should be as low as possible and *R* as high. According to all these, it is evaluated that using the ECG signal and the GPR algorithm, and BP detection can be performed in 16 seconds in the minimum desired time.

The tabular models defined for SBP apply to DBP. The tables for the whole process are modeled separately (Tables 14–23). Models using all feature groups obtained the best performance value for each epoched period. Accordingly, DBP of MAPE = 3.31 mmHg and 0.97 mmHg for 2 seconds were obtained using the EBT algorithm (Table 14). DBP values of MAPE = 3.17 mmHg and 0.97 mmHg for the 4 seconds were obtained using the EBT algorithm (Table 15). DBP values of MAPE = 3.14 mmHg and 0.97 mmHg for 6 seconds were obtained using the EBT algorithm (Table 16). DBP values of MAPE = 3.11 mmHg and 0.97 mmHg for 8 seconds were obtained using the EBT algorithm (Table 17). DBP values of MAPE = 2.69 mmHg and 0.97 mmHg for 10 seconds were obtained using the EBT algorithm (Table 18). DBP values of MAPE = 2.88 mmHg and 0.97 mmHg for the 12 seconds were obtained using the GP algorithm (Table 19). DBP values of MAPE = 3.28 mmHg and 0.98 mmHg for 14 seconds were obtained using the EBT algorithm (Table 20). DBP values of MAPE = 2.44 mmHg and 0.98 mmHg for 16 seconds were obtained using the GPR algorithm (Table 21). DBP values MAPE = 2.49 mmHg and 0.97 mmHg for the 18 seconds were obtained using the EBT algorithm (Table 22). DBP values of MAPE = 2.37 mmHg and 0.97 mmHg for the 20 seconds were obtained using the EBT algorithm (Table 23).

The performance tables of the models created for DBP prediction should be carefully examined. For each increasing epoch time, both decreases and increases in MAPE were observed together, and the lowest MAPE value was obtained in Table 23. Accordingly, considering the *R* value, the maximum value was obtained in Tables 20 and 21. It is desirable for MAPE to be as low as possible and *R* high. According to all these, it is evaluated that DBP detection can be performed in 16 seconds using the ECG signal and the GPR algorithm in the minimum desired time. A 0.07 drop-in MAPE for 20 seconds is not very significant. For this reason, 16 seconds is considered suitable for time determination. Also, the summarized pattern table for the whole process is given in Table 24. In addition to all these, the GPR algorithm is evaluated to be appropriate for SBP and DBP time detection since it fits well with the ECG-based dataset.

Bland-Altman plots were prepared for the proposed models (Figure 4). It was determined that the resulting error rates of the models were close to zero, and the correlation values were *R* = 0.97 (Table 23). The difference between the actual and predicted values is expected to be zero. Each scatter being close to zero indicates good performance.

The best findings obtained in the study were compared with literature studies (Table 23). The findings show that the proposed models are compatible with the literature and are a step forward in performance and low processing time.

## 4. Discussions

Since hypertension is known as a silent killer, patients with hypertension should be followed constantly [1, 3]. In order to keep hypertension under control, patients are expected to strictly comply with drug treatments [3]. There is a need for new technologies that can be used without the need for technical knowledge for continuous monitoring of hypertension at home [2, 3]. This study is aimed at calculating the ECG signal and machine learning-based minimum BP time response in hypertension patients. First, ECG signal data of five individuals were collected in the study. The signals were then divided into periods of 2-4-6-8-10-12-14-16-18-20 seconds. 25 statistical features in the time domain were extracted from each epoched signal. The feature selection algorithm is used to reduce the model's unnecessary workload and provide size optimization. With EBT, GPR, and FT algorithms, selected features were used for BP estimation. BP estimation performance values for each epoched period were calculated within certain characteristics and recorded in tables (Tables 4–23). According to these tables, BP estimation can be evaluated at a minimum time. The model proposed in the study differs significantly from the studies in the literature in terms of time epoching. BP calculation was performed for each period. Calculated BP values exhibited a unique structure at each step and increased performance. After first determining the statistical inputs for the ECG signal, it was determined that the model's performance was low against some features. On the other hand, unnecessary features were removed by optimizing the size. In this way, the performance increase was observed on datasets with high correlation levels. In this system, which tried to be improved gradually, periodic observations were made graphically, and minimum time detection was achieved with a high accuracy rate. The proposed model is among the algorithms with high accuracy obtained in the literature so far (Table 23, *R* = 0.98 mmHg).

The most striking feature of the study is that it detects BP values for each period by epoching the ECG signal. Research on ECG, PPG, and BP properties is carried out extensively in the literature [31, 33, 78]. Among these signals, QRS and other components exhibited in a heartbeat in the ECG signal, which is the research subject of the study, are generally preferred as feature input [27, 33, 34]. Due to changes in the ECG signal, feature extraction can cause workload and computational complexity. On the other hand, statistical parameters were used, and BP estimation performance evaluation was made on epoched ECG signals. The best performance value that can be calculated in minimum time is *R* = 0.98 (Table 24, 16 seconds). It is understood that BP can be detected with high accuracy for two seconds, and applications can be performed within this period. The study used the 16-second epoched signal model for BP estimation. This is because we can reduce the error rate and see the minimum and maximum points in an epoch. ECG and BP are similar signals. The averages of the BP signal's local minimum points and local maximum points correspond to the DBP and SBP values, respectively. The multiplicity of these points reduces the error rate and increases the execution time. In this condition, the design was realized. In the literature studies, no research has yet been carried out to determine BP in a certain period. Although the article has an original research topic, it has the infrastructure to answer new research questions. Accordingly, with how many seconds of ECG recording can a highly accurate BP prediction model be developed? The study findings show that BP estimation can be made with an ECG signal with at least two-second epochs. However, the highest performance was achieved in the 16-second epoch, but the performance change is not appreciable. For this reason, it is considered that high performance can be obtained from two-second epochs with different signal processing processes.

The datasets are summarized significantly with the help of descriptive statistical parameters. In this study, the ECG signal with 25 feature sets was converted to a clearer dataset (Table 2). Studies in the literature are often based on specific characteristics [31, 33, 34]. In addition, temporal, chaotic, and morphological features are most well-liked in deep learning-based studies [20, 34]. However, studies based on different feature extraction algorithms seem to be insufficient in terms of performance (Table 25) [27, 29]. In this respect, it can be considered that the feature extraction algorithm used in the study has a better structure compared to the literature.

The feature selection process with classical machine learning methods is recommended. However, this process has not been applied in many BP estimation studies [28, 31, 33]. The feature selection algorithm performed better than the literature by optimizing the size of the model used and eliminating unnecessary features.

EBT, GPR, and FT algorithms in the proposed model have been an important element in determining model performance. The performance values of these models on each epoched signal show how compatible that algorithm is with the epoched dataset. This situation indicates that there is algorithm variation between epoched signals in Table 24. The proposed models are one step ahead of the studies in the literature in terms of performance (Table 25).

### 4.1. Strengths and Limitations

The use of machine learning algorithms in terms of continuous cuffless BP estimation, feature extraction, and evaluation processes that do not require calibration is still a matter of debate for accurate diagnosis and treatment. This study compares their performance using various ML techniques. Statistical feature extraction was applied from each epoched signal by applying the epoching process to the ECG signals. The dataset in which ML techniques were evaluated showed high performance for each epoch. Although different feature sets have been extracted for the model, the morphological features of the ECG signal have not been investigated. In addition, increasing the demographic information of the subjects can improve the BP prediction performance. Even if there are technical failures in the collection of the dataset, the operations applied to the signal in the software environment prevent this data loss, and its effect on performance is minimized.

## 5. Conclusions

Monitoring of BP is vital for the follow-up and treatment of hypertension. Algorithms and devices that comply with new reliable standards are needed for home BP monitoring. These technologies are expected to offer effortless measurement. This study developed artificial intelligence-based algorithms to monitor BP with ECG. The study's main question is “What is the minimum time required for BP determination by ECG?” For this purpose, models have been developed for signals with different durations between 2 and 20 seconds, and algorithms have been tested.

It has been determined that BP estimation can be made with high accuracy for any time including 2 seconds. While *R* = 0.98 for 14- and 16-second epochs, it was determined as *R* = 0.97 for 2-second epoch. It varies in the range of 0.97 ≤ *R*≤ 0.98 in other periods. This sitution indicates that BP can be detected with high accuracy for ECG.

The innovations included in the findings of this study are as follows. (1) With ECG, BP can be predicted accurately. (2) Shortening the ECG signal time does not affect the success rate. (3) BP can be estimated with a 2-second epoch. (4) Feature extraction and selection processes improved model performance. (5) Artificial intelligence-based models have increased system reliability. Due to the high performance and reliability of the proposed model, it is considered that it can be used as an auxiliary software for BP monitoring in all systems that can measure ECG signals.

## 6. Future Work

With these encouraging results, future studies are planned. The scope of the study can be expanded by using a dataset containing many diverse groups of people and more specific ML techniques. Increasing the sampling frequency of the signals will prevent information loss. For this reason, a sampling frequency of at least 2.5 times the signal frequency range is recommended for new studies. In addition, studies can be continued by looking at the relationship between ECG and BP from another perspective by considering the morphological features of the ECG signal and extracting the frequency domain feature groups on the dataset.

## Figures and Tables

**Figure 1:** Application flowchart.

**Figure 2:** Sample diary records.

**Figure 3:** Calculation of BP values for the 4-second sample.

**Figure 4:** Blant-Altman plots for proposed (a) DBP and (b) SBP models.

**Table 1:** Representation of features mathematical and code.

Nu	Feature	Equation
1	Kurtosis	$x_{\text{kur}}=\frac{\sum_{i=1}^{n}{\left(x\left(i\right)-\overset{¯}{x}\right)}^{4}}{\left(n-1\right)S^{4}}$
2	Skewness	$x_{\text{ske}}=\frac{\sum_{i=1}^{n}{\left(x_{i}-\overset{¯}{x}\right)}^{3}}{\left(n-1\right)S^{3}}$
3	∗IQR	IQR = iqr(*x*)
4	CV	$\text{CV}=\left(\frac{S}{\overset{¯}{x}}\right)100$
5	Geometric mean	$G=\sqrt[{n}]{x_{1}+\cdots +x_{n}}$
6	Harmonic mean	$H=\frac{n}{\left(1/x_{1}\right)+\cdots +\left(1/x_{n}\right)}$
7	Activity-Hjort parameters	*A* = *S*^2^
8	Mobility-Hjort parameters	$M=\frac{S_{1}^{2}}{S^{2}}$
9	Complexity-Hjort parameters	$C=\sqrt{{\left(\frac{S_{2}^{2}}{S_{1}^{2}}\right)}^{2}-{\left(\frac{S_{1}^{2}}{S^{2}}\right)}^{2}}$
10	∗Maximum	*x*_max_ = max(*x*_*i*_)
11	Median	$\overset{\sim }{x}=\left\{\begin{array}{cc} x_{\left(\left(n+1\right)/2\right)} & :x\text{ odd}\\ \frac{1}{2}\left(x_{n/2}+x_{\left(n/2\right)+1}\right) & :x\text{ even} \end{array}\right.$
12	^∗^Mean absolute deviation	MAD = mad(*x*)
13	∗Minimum	*x*_min_ = min(*x*_*i*_)
14	∗Central moments	CM = moment(*x*, 10)
15	Mean	$\overset{¯}{x}=\frac{1}{n}\overset{n}{\underset{i=1}{\sum }}=\frac{1}{n}\left(x_{1}+\cdots +x_{n}\right)$
16	Average curve length	$\text{CL}=\frac{1}{n}\overset{n}{\underset{i=2}{\sum }}\left|x_{i}-x_{i-1}\right|$
17	Average energy	$E=\frac{1}{n}\overset{n}{\underset{i=1}{\sum }}x_{i}^{2}$
18	Root mean squared	$X_{\text{rms}}=\sqrt{\frac{1}{n}\overset{n}{\underset{i=1}{\sum }}{\left|x_{i}\right|}^{2}}$
19	Standard error	$S_{\overset{¯}{x}}=\frac{S}{\sqrt{n}}$
20	Standard deviation	$S=\sqrt{\frac{1}{n}\overset{n}{\underset{i=1}{\sum }}\left(x_{i}-\overset{¯}{x}\right)}$
21	Shape factor	$\text{SF}=\frac{X_{\text{rms}}}{1/n\sum_{i=1}^{n}\sqrt{\left|x_{i}\right|}}$
22	∗Singular value decomposition	SVD = svd(*x*)
23	∗ 25% trimmed mean	*T*25 = trimmean(*x*, 25)
24	∗ 50% trimmed mean	*T*50 = trimmean(*x*, 50)
25	Average Teager energy	$\text{TE}=\frac{1}{n}\overset{n}{\underset{i=3}{\sum }}\left(x_{i-1}^{2}-x_{i}x_{i-2}\right)$

∗ The property was computed using MATLAB. IQR: interquartile range; CV: coefficient of variation. *S*^2^: variance of the signal *x*. *S*_1_^2^: variance of the 1st derivative of the signal *x*. *S*_2_^2^: variance of the 2nd derivative of the signal *x*.

**Table 2:** Spearman's correlation coefficient for each extracted feature set.

Info		Spearman's correlation coefficient for each extracted feature set																								
R	BP	25	24	23	22	21	20	19	18	17	16	15	14	13	12	11	10	9	8	7	6	5	4	3	2	1
2	SBP	0.12	0.02	0.02	0.09	**0.66**	0.22	0.18	0.09	0.09	0.10	0.06	0.23	0.06	0.23	0.15	0.22	0.22	0.22	0.22	0.00	0.03	0.22	0.18	0.15	0.02
	DBP	0.12	0.02	0.02	0.09	**0.66**	0.22	0.18	0.09	0.09	0.10	0.06	0.23	0.06	0.23	0.15	0.22	0.22	0.22	0.22	0.00	0.03	0.22	0.18	0.15	0.02
4	SBP	0.17	0.02	0.04	0.18	**0.65**	0.24	0.21	0.18	0.18	0.48	0.14	0.26	0.09	0.23	0.16	0.24	0.24	0.24	0.24	0.02	0.08	0.24	0.19	0.20	0.00
	DBP	0.17	0.02	0.04	0.18	**0.65**	0.24	0.21	0.18	0.18	0.48	0.14	0.26	0.09	0.23	0.16	0.24	0.24	0.24	0.24	0.02	0.08	0.24	0.19	0.20	0.00
6	SBP	0.20	0.03	0.06	0.26	**0.67**	0.24	0.22	0.26	0.26	0.18	0.20	0.26	0.10	0.22	0.17	0.24	0.24	0.24	0.24	0.03	0.12	0.24	0.19	0.22	0.00
	DBP	0.20	0.03	0.06	0.26	**0.67**	0.24	0.22	0.26	0.26	0.18	0.20	0.26	0.10	0.22	0.17	0.24	0.24	0.24	0.24	0.03	0.12	0.24	0.19	0.22	0.00
8	SBP	0.21	0.04	0.06	0.30	**0.68**	0.24	0.22	0.30	0.30	0.36	0.25	0.26	0.11	0.22	0.17	0.24	0.24	0.24	0.24	0.02	0.14	0.24	0.20	0.23	0.01
	DBP	0.21	0.04	0.06	0.30	**0.68**	0.24	0.22	0.30	0.30	0.36	0.25	0.26	0.11	0.22	0.17	0.24	0.24	0.24	0.24	0.02	0.14	0.24	0.20	0.23	0.01
10	SBP	0.21	0.04	0.07	0.34	**0.68**	0.24	0.22	0.34	0.34	0.07	0.30	0.26	0.11	0.21	0.17	0.23	0.24	0.24	0.24	0.02	0.16	0.24	0.20	0.23	0.01
	DBP	0.21	0.04	0.07	0.34	**0.68**	0.24	0.22	0.34	0.34	0.07	0.30	0.26	0.11	0.21	0.17	0.23	0.24	0.24	0.24	0.02	0.16	0.24	0.20	0.23	0.01
12	SBP	0.22	0.04	0.07	0.37	**0.69**	0.24	0.22	0.37	0.37	0.27	0.34	0.26	0.12	0.21	0.17	0.23	0.24	0.24	0.24	0.02	0.18	0.24	0.21	0.24	0.02
	DBP	0.22	0.04	0.07	0.37	**0.69**	0.24	0.22	0.37	0.37	0.27	0.34	0.26	0.12	0.21	0.17	0.23	0.24	0.24	0.24	0.02	0.18	0.24	0.21	0.24	0.02
14	SBP	0.22	0.04	0.08	0.39	**0.92**	0.24	0.22	0.39	0.39	0.11	0.38	0.26	0.12	0.21	0.17	0.23	0.24	0.24	0.24	0.02	0.19	0.24	0.21	0.24	0.02
	DBP	0.22	0.04	0.08	0.39	**0.92**	0.24	0.22	0.39	0.39	0.11	0.38	0.26	0.12	0.21	0.17	0.23	0.24	0.24	0.24	0.02	0.19	0.24	0.21	0.24	0.02
**16**	**SBP**	0.23	0.04	0.08	0.39	**0.93**	0.24	0.23	0.39	0.39	0.10	0.41	0.26	0.12	0.21	0.17	0.23	0.24	0.24	0.24	0.02	0.20	0.24	0.22	0.24	0.02
	**DBP**	0.23	0.04	0.08	0.39	**0.93**	0.24	0.23	0.39	0.39	0.10	0.41	0.26	0.12	0.21	0.17	0.23	0.24	0.24	0.24	0.02	0.20	0.24	0.22	0.24	0.02
18	SBP	0.23	0.04	0.08	0.41	**0.70**	0.24	0.23	0.41	0.41	0.51	0.44	0.26	0.12	0.21	0.18	0.23	0.24	0.24	0.24	0.01	0.22	0.24	0.22	0.24	0.02
	DBP	0.23	0.04	0.08	0.41	**0.70**	0.24	0.23	0.41	0.41	0.51	0.44	0.26	0.12	0.21	0.18	0.23	0.24	0.24	0.24	0.01	0.22	0.24	0.22	0.24	0.02
20	SBP	0.23	0.04	0.08	0.41	**0.70**	0.24	0.23	0.41	0.41	0.12	0.46	0.26	0.13	0.21	0.18	0.23	0.24	0.24	0.24	0.02	0.22	0.24	0.22	0.24	0.02
	DBP	0.23	0.04	0.08	0.41	**0.70**	0.24	0.23	0.41	0.41	0.12	0.46	0.26	0.13	0.21	0.18	0.23	0.24	0.24	0.24	0.02	0.22	0.24	0.22	0.24	0.02

R: rank; BP: blood pressure; SBP: systolic blood pressure; DBP: diastolic blood pressure.

**Table 3:** Distribution of training and testing data.

Dataset	Train (%80)	Test (%20)	Total
Diastolic	3866	966	4832
Systolic	3866	966	4832

**Table 4:** SBP prediction models for 2-second epoching.

Info				Performance evaluation criteria						
L	FN	FP	Model	MAPE	MAD	SE	MSE	RMSE	*R*	*R* ^2^
1	1	5	FT	7.15	9.10	11.79	138.93	11.79	0.62	0.39
			GPR	6.24	7.91	10.00	99.97	10.00	0.66	0.44
			EBT	6.54	8.30	10.62	112.75	10.62	0.64	0.41

2	3	10	FT	5.38	6.92	10.04	100.83	10.04	0.79	0.62
			GPR	6.31	7.99	9.99	99.84	9.99	0.66	0.44
			EBT	4.64	5.95	8.33	69.45	8.33	0.83	0.69

3	4	15	FT	5.11	6.58	9.74	94.86	9.74	0.81	0.66
			GPR	5.05	6.45	8.63	74.44	8.63	0.82	0.67
			EBT	4.37	5.62	7.94	63.10	7.94	0.85	0.73

4	5	20	FT	5.11	6.58	9.74	94.86	9.74	0.81	0.66
			GPR	4.99	6.38	8.57	73.49	8.57	0.82	0.67
			EBT	4.35	5.59	7.91	62.58	7.91	0.86	0.73

5	6	25	FT	5.19	6.68	9.85	97.07	9.85	0.81	0.65
			GPR	5.00	6.39	8.58	73.60	8.58	0.82	0.67
			EBT	4.39	5.63	7.96	63.41	7.96	0.85	0.73

6	8	30	FT	5.20	6.69	9.87	97.46	9.87	0.81	0.65
			GPR	4.93	6.30	8.52	72.49	8.51	0.82	0.68
			EBT	4.37	5.61	7.91	62.57	7.91	0.86	0.73

7	9	35	FT	4.66	6.01	9.01	81.15	9.01	0.85	0.72
			GPR	4.64	5.93	8.18	66.86	8.18	0.84	0.71
			EBT	4.12	5.29	7.52	56.47	7.51	0.88	0.77

8	10	40	FT	4.22	5.47	8.25	68.11	8.25	0.88	0.78
			GPR	4.10	5.28	7.32	53.54	7.32	0.88	0.78
			EBT	3.73	4.82	6.90	47.54	6.89	0.90	0.81

9	11	45	FT	4.22	5.48	8.26	68.14	8.25	0.88	0.78
			GPR	4.12	5.31	7.34	53.92	7.34	0.88	0.78
			EBT	3.77	4.87	6.96	48.40	6.96	0.90	0.81

10	13	50	FT	3.24	4.24	6.44	41.41	6.43	0.95	0.90
			GPR	2.86	3.73	5.39	29.06	5.39	0.96	0.92
			EBT	2.76	3.60	5.32	28.29	5.32	0.96	0.92

11	25	100	FT	3.19	4.16	6.49	42.12	6.49	0.95	0.91
			GPR	2.68	3.49	5.12	26.18	5.12	0.97	0.93
			EBT	**2.58**	**3.37**	**5.05**	**25.48**	**5.05**	**0.97**	**0.93**

L: level; FN: number of feature; FP: percentage of feature; FT: fine tree; GPR: Gaussian process regression; EBT: ensemble bagged tree.

**Table 5:** SBP prediction models for 4-second epoching.

Info				Performance evaluation criteria						
L	FN	FP	Model	MAPE	MAD	SE	MSE	RMSE	*R*	*R* ^2^
1	1	5	FT	6.54	8.45	11.24	126.33	11.24	0.63	0.40
			GPR	5.86	7.55	9.73	94.61	9.73	0.66	0.43
			EBT	6.09	7.85	10.30	106.13	10.30	0.64	0.41

2	3	10	FT	3.83	5.01	7.40	54.74	7.40	0.92	0.85
			GPR	4.09	5.28	7.30	53.20	7.29	0.91	0.82
			EBT	3.22	4.20	6.20	38.43	6.20	0.94	0.87

3	4	15	FT	3.60	4.73	7.14	50.94	7.14	0.93	0.86
			GPR	3.27	4.28	6.31	39.83	6.31	0.93	0.86
			EBT	3.04	3.99	5.94	35.24	5.94	0.94	0.89

4	5	20	FT	3.60	4.73	7.14	50.94	7.14	0.93	0.86
			GPR	3.28	4.29	6.30	39.73	6.30	0.93	0.86
			EBT	3.04	3.99	5.94	35.21	5.93	0.94	0.88

5	6	25	FT	3.63	4.77	7.22	52.07	7.22	0.93	0.86
			GPR	3.27	4.28	6.30	39.67	6.30	0.93	0.86
			EBT	3.07	4.02	5.97	35.61	5.97	0.94	0.88

6	8	30	FT	3.63	4.77	7.25	52.50	7.25	0.93	0.86
			GPR	3.26	4.27	6.29	39.56	6.29	0.93	0.86
			EBT	3.05	4.01	5.96	35.53	5.96	0.94	0.89

7	9	35	FT	3.56	4.68	7.09	50.19	7.08	0.93	0.86
			GPR	3.09	4.04	6.05	36.58	6.05	0.94	0.88
			EBT	3.00	3.94	5.89	34.64	5.89	0.94	0.89

8	10	40	FT	3.38	4.45	6.86	47.00	6.86	0.94	0.87
			GPR	2.93	3.84	5.80	33.67	5.80	0.94	0.89
			EBT	2.85	3.75	5.68	32.30	5.68	0.95	0.90

9	11	45	FT	3.38	4.45	6.86	47.00	6.86	0.94	0.87
			GPR	2.90	3.80	5.78	33.39	5.78	0.95	0.89
			EBT	2.83	3.72	5.63	31.65	5.63	0.95	0.90

10	13	50	FT	2.98	3.95	6.21	38.55	6.21	0.96	0.92
			GPR	2.53	3.33	5.03	25.25	5.02	0.96	0.93
			EBT	2.53	3.34	5.08	25.83	5.08	0.96	0.93

11	25	100	FT	2.82	3.72	5.92	35.01	5.92	0.96	0.92
			GPR	2.42	3.18	4.89	23.91	4.89	0.97	0.94
			EBT	**2.34**	**3.09**	**4.86**	**23.62**	**4.86**	**0.97**	**0.94**

L: level; FN: number of feature; FP: percentage of feature; FT: fine tree; GPR: Gaussian process regression; EBT: ensemble bagged tree.

**Table 6:** SBP prediction models for 6-second epoching.

Info				Performance evaluation criteria						
L	FN	FP	Model	MAPE	MAD	SE	MSE	RMSE	*R*	*R* ^2^
1	1	5	FT	6.31	8.19	11.09	122.81	11.08	0.65	0.42
			GPR	5.58	7.22	9.52	90.49	9.51	0.70	0.49
			EBT	5.87	7.60	10.14	102.83	10.14	0.67	0.44

2	3	10	FT	5.11	6.68	9.80	95.97	9.80	0.79	0.62
			GPR	5.68	7.34	9.56	91.31	9.56	0.70	0.49
			EBT	4.63	6.01	8.39	70.43	8.39	0.82	0.68

3	4	15	FT	5.11	6.67	9.79	95.81	9.79	0.79	0.62
			GPR	5.67	7.33	9.56	91.24	9.55	0.70	0.50
			EBT	4.58	5.94	8.36	69.83	8.36	0.83	0.68

4	5	20	FT	5.11	6.67	9.79	95.81	9.79	0.79	0.62
			GPR	5.67	7.34	9.56	91.27	9.55	0.70	0.49
			EBT	4.59	5.97	8.38	70.12	8.37	0.82	0.68

5	6	25	FT	5.08	6.64	9.89	97.72	9.89	0.79	0.62
			GPR	5.07	6.56	8.97	80.47	8.97	0.78	0.61
			EBT	4.46	5.79	8.23	67.75	8.23	0.83	0.70

6	8	30	FT	5.08	6.64	9.89	97.79	9.89	0.79	0.62
			GPR	4.99	6.45	8.89	79.01	8.89	0.78	0.61
			EBT	4.45	5.79	8.22	67.58	8.22	0.83	0.70

7	9	35	FT	5.03	6.58	9.80	96.04	9.80	0.79	0.62
			GPR	4.97	6.44	8.88	78.79	8.88	0.78	0.61
			EBT	4.43	5.77	8.22	67.52	8.22	0.83	0.70

8	10	40	FT	5.05	6.61	9.80	95.97	9.80	0.79	0.63
			GPR	4.97	6.44	8.88	78.77	8.88	0.78	0.61
			EBT	4.45	5.80	8.28	68.56	8.28	0.83	0.69

9	11	45	FT	4.59	6.01	9.23	85.13	9.23	0.83	0.70
			GPR	4.80	6.20	8.57	73.41	8.57	0.81	0.65
			EBT	4.19	5.45	7.85	61.59	7.85	0.86	0.74

10	13	50	FT	2.98	3.95	6.27	39.31	6.27	0.95	0.91
			GPR	2.62	3.47	5.28	27.87	5.28	0.96	0.92
			EBT	2.57	3.41	5.26	27.61	5.25	0.96	0.92

11	25	100	FT	2.73	3.61	6.06	36.68	6.06	0.96	0.92
			GPR	2.36	3.13	4.94	24.41	4.94	0.97	0.94
			EBT	**2.27**	**3.00**	**4.83**	**23.31**	**4.83**	**0.97**	**0.94**

L: level; FN: number of feature; FP: percentage of feature; FT: fine tree; GPR: Gaussian process regression; EBT: ensemble bagged tree.

**Table 7:** SBP prediction models for 8-second epoching.

Info				Performance evaluation criteria						
L	FN	FP	Model	MAPE	MAD	SE	MSE	RMSE	*R*	*R* ^2^
1	1	5	FT	5.88	7.69	10.61	112.46	10.60	0.68	0.46
			GPR	5.31	6.92	9.08	82.35	9.07	0.73	0.54
			EBT	5.53	7.20	9.67	93.48	9.67	0.71	0.50

2	3	10	FT	4.49	5.91	8.75	76.48	8.75	0.84	0.71
			GPR	5.20	6.76	8.93	79.66	8.93	0.77	0.59
			EBT	4.49	5.85	8.09	65.43	8.09	0.84	0.70

3	4	15	FT	4.49	5.91	8.75	76.54	8.75	0.84	0.71
			GPR	5.20	6.77	8.94	79.82	8.93	0.76	0.58
			EBT	4.45	5.80	8.05	64.72	8.05	0.84	0.71

4	5	20	FT	4.49	5.91	8.75	76.54	8.75	0.84	0.71
			GPR	5.20	6.77	8.95	80.04	8.95	0.76	0.58
			EBT	4.52	5.89	8.19	67.03	8.19	0.83	0.69

5	6	25	FT	4.50	5.90	8.91	79.40	8.91	0.84	0.70
			GPR	5.20	6.77	8.95	80.02	8.95	0.76	0.58
			EBT	4.14	5.39	7.63	58.12	7.62	0.86	0.74

6	8	30	FT	4.66	6.09	9.23	85.13	9.23	0.82	0.67
			GPR	4.72	6.15	8.44	71.21	8.44	0.81	0.65
			EBT	3.98	5.20	7.49	56.01	7.48	0.87	0.76

7	9	35	FT	4.66	6.09	9.23	85.13	9.23	0.82	0.67
			GPR	4.67	6.08	8.36	69.77	8.35	0.81	0.66
			EBT	3.97	5.19	7.50	56.13	7.49	0.87	0.75

8	10	40	FT	4.70	6.15	9.26	85.72	9.26	0.82	0.67
			GPR	4.61	6.01	8.29	68.67	8.29	0.82	0.67
			EBT	3.97	5.19	7.48	55.87	7.47	0.87	0.76

9	11	45	FT	4.68	6.13	9.19	84.31	9.18	0.82	0.68
			GPR	4.60	6.00	8.28	68.47	8.27	0.82	0.67
			EBT	3.98	5.20	7.51	56.32	7.50	0.87	0.75

10	13	50	FT	4.48	5.87	8.97	80.37	8.96	0.85	0.72
			GPR	4.41	5.74	8.01	64.18	8.01	0.84	0.70
			EBT	3.83	5.01	7.24	52.37	7.24	0.88	0.78

11	25	100	FT	2.54	3.37	5.71	32.62	5.71	0.96	0.93
			GPR	**2.20**	**2.91**	**4.50**	**20.28**	**4.50**	**0.97**	**0.95**
			EBT	2.13	2.81	4.56	20.74	4.55	0.97	0.95

L: level; FN: number of feature; FP: percentage of feature; FT: fine tree; GPR: Gaussian process regression; EBT: ensemble bagged tree.

**Table 8:** SBP prediction models for 10-second epoching.

Info				Performance evaluation criteria						
L	FN	FP	Model	MAPE	MAD	SE	MSE	RMSE	*R*	*R* ^2^
1	1	5	FT	5.68	7.42	10.29	105.82	10.29	0.71	0.50
			GPR	5.17	6.74	8.85	78.30	8.85	0.75	0.57
			EBT	5.31	6.92	9.37	87.64	9.36	0.73	0.53

2	3	10	FT	5.10	6.68	9.91	98.04	9.90	0.77	0.59
			GPR	5.08	6.63	8.75	76.43	8.74	0.76	0.58
			EBT	4.73	6.16	8.59	73.71	8.59	0.81	0.65

3	4	15	FT	5.10	6.68	9.91	98.04	9.90	0.77	0.59
			GPR	5.07	6.62	8.74	76.39	8.74	0.76	0.58
			EBT	4.66	6.08	8.57	73.33	8.56	0.81	0.65

4	5	20	FT	5.09	6.66	9.91	98.20	9.91	0.77	0.60
			GPR	4.91	6.39	8.66	74.92	8.66	0.78	0.61
			EBT	4.57	5.97	8.50	72.24	8.50	0.81	0.66

5	6	25	FT	4.57	5.97	9.03	81.45	9.02	0.83	0.68
			GPR	4.91	6.39	8.66	74.92	8.66	0.78	0.61
			EBT	4.13	5.39	7.73	59.69	7.73	0.86	0.73

6	8	30	FT	4.59	5.99	9.13	83.22	9.12	0.83	0.68
			GPR	4.46	5.82	8.15	66.38	8.15	0.83	0.68
			EBT	4.01	5.22	7.70	59.19	7.69	0.86	0.74

7	9	35	FT	4.56	5.96	9.11	82.98	9.11	0.83	0.68
			GPR	4.46	5.81	8.15	66.28	8.14	0.83	0.68
			EBT	3.99	5.21	7.67	58.82	7.67	0.86	0.74

8	10	40	FT	4.60	6.02	9.14	83.52	9.14	0.82	0.68
			GPR	4.47	5.82	8.15	66.39	8.15	0.83	0.68
			EBT	4.01	5.23	7.70	59.23	7.70	0.86	0.74

9	11	45	FT	4.60	6.01	9.14	83.39	9.13	0.82	0.68
			GPR	4.44	5.79	8.14	66.20	8.14	0.83	0.68
			EBT	3.99	5.21	7.68	58.85	7.67	0.86	0.74

10	13	50	FT	2.97	3.93	6.07	36.86	6.07	0.95	0.90
			GPR	2.66	3.51	5.17	26.75	5.17	0.96	0.91
			EBT	2.58	3.41	5.14	26.39	5.14	0.96	0.92

11	25	100	FT	2.40	3.21	5.44	29.60	5.44	0.97	0.93
			GPR	2.17	2.88	4.50	20.27	4.50	0.97	0.95
			EBT	**2.08**	**2.75**	**4.37**	**19.11**	**4.37**	**0.97**	**0.95**

L: level; FN: number of feature; FP: percentage of feature; FT: fine tree; GPR: Gaussian process regression; EBT: ensemble bagged tree.

**Table 9:** SBP prediction models for 12-second epoching.

Info				Performance evaluation criteria						
L	FN	FP	Model	MAPE	MAD	SE	MSE	RMSE	*R*	*R* ^2^
1	1	5	FT	5.45	7.18	10.02	100.18	10.01	0.71	0.51
			GPR	4.95	6.46	8.61	73.99	8.60	0.77	0.60
			EBT	5.10	6.70	9.11	82.95	9.11	0.74	0.55

2	3	10	FT	4.67	6.18	9.16	83.80	9.15	0.81	0.65
			GPR	4.76	6.25	8.37	69.95	8.36	0.79	0.62
			EBT	4.28	5.60	7.95	63.19	7.95	0.84	0.71

3	4	15	FT	4.67	6.18	9.16	83.80	9.15	0.81	0.65
			GPR	4.76	6.25	8.38	70.11	8.37	0.79	0.62
			EBT	4.21	5.50	7.92	62.60	7.91	0.84	0.71

4	5	20	FT	4.64	6.12	9.01	81.00	9.00	0.81	0.66
			GPR	4.53	5.94	8.21	67.28	8.20	0.81	0.65
			EBT	4.13	5.42	7.83	61.28	7.83	0.84	0.71

5	6	25	FT	4.21	5.57	8.32	69.10	8.31	0.87	0.75
			GPR	3.80	5.01	7.20	51.76	7.19	0.87	0.77
			EBT	3.73	4.90	7.07	49.98	7.07	0.89	0.79

6	8	30	FT	3.79	5.01	7.83	61.25	7.83	0.89	0.79
			GPR	3.58	4.73	6.95	48.30	6.95	0.89	0.79
			EBT	3.35	4.40	6.58	43.26	6.58	0.91	0.83

7	9	35	FT	3.79	5.01	7.83	61.25	7.83	0.89	0.79
			GPR	3.56	4.70	6.89	47.38	6.88	0.89	0.79
			EBT	3.35	4.39	6.61	43.65	6.61	0.91	0.83

8	10	40	FT	3.80	5.02	7.84	61.44	7.84	0.89	0.78
			GPR	3.56	4.70	6.88	47.29	6.88	0.89	0.79
			EBT	3.34	4.39	6.58	43.26	6.58	0.91	0.83

9	11	45	FT	3.80	5.02	7.85	61.48	7.84	0.89	0.78
			GPR	3.56	4.71	6.87	47.07	6.86	0.89	0.79
			EBT	3.31	4.35	6.51	42.26	6.50	0.91	0.83

10	13	50	FT	2.94	3.91	6.09	37.06	6.09	0.95	0.90
			GPR	2.73	3.65	5.31	28.18	5.31	0.95	0.91
			EBT	2.58	3.42	5.16	26.57	5.15	0.96	0.92

11	25	100	FT	2.38	3.19	5.53	30.51	5.52	0.97	0.93
			GPR	**2.04**	**2.73**	**4.39**	**19.25**	**4.39**	**0.98**	**0.95**
			EBT	2.05	2.73	4.46	19.90	4.46	0.98	0.95

L: level; FN: number of feature; FP: percentage of feature; FT: fine tree; GPR: Gaussian process regression; EBT: ensemble bagged tree.

**Table 10:** SBP prediction models for 14-second epoching.

Info				Performance evaluation criteria						
L	FN	FP	Model	MAPE	MAD	SE	MSE	RMSE	*R*	*R* ^2^
1	1	5	FT	3.56	4.75	6.42	41.10	6.41	0.92	0.84
			GPR	3.02	4.02	5.39	29.00	5.39	0.94	0.87
			EBT	3.31	4.41	5.90	34.81	5.90	0.92	0.85

2	3	10	FT	3.23	4.33	6.12	37.41	6.12	0.94	0.88
			GPR	3.28	4.38	12.62	159.13	12.61	0.94	0.88
			EBT	2.96	3.91	5.70	32.48	5.70	0.94	0.89

3	4	15	FT	3.23	4.33	6.12	37.41	6.12	0.94	0.88
			GPR	3.73	5.01	27.49	754.77	27.47	0.94	0.88
			EBT	2.88	3.82	5.44	29.54	5.44	0.94	0.89

4	5	20	FT	3.18	4.28	6.06	36.63	6.05	0.94	0.89
			GPR	4.97	6.77	105.52	11118.50	105.44	0.95	0.90
			EBT	2.85	3.78	5.43	29.41	5.42	0.95	0.90

5	6	25	FT	3.01	4.02	5.91	34.90	5.91	0.95	0.90
			GPR	3.58	4.83	30.51	929.23	30.48	0.95	0.90
			EBT	2.72	3.58	5.35	28.60	5.35	0.96	0.91

6	8	30	FT	2.93	3.91	5.99	35.81	5.98	0.95	0.91
			GPR	5.40	7.36	117.78	13851.43	117.69	0.95	0.90
			EBT	2.59	3.43	5.06	25.61	5.06	0.96	0.92

7	9	35	FT	2.93	3.91	5.99	35.81	5.98	0.95	0.91
			GPR	3.97	5.22	7.43	55.09	7.42	0.86	0.75
			EBT	2.61	3.45	5.11	26.03	5.10	0.96	0.92

8	10	40	FT	2.92	3.90	5.96	35.48	5.96	0.95	0.91
			GPR	4.96	6.72	101.53	10293.64	101.46	0.95	0.90
			EBT	2.61	3.46	5.13	26.25	5.12	0.96	0.92

9	11	45	FT	2.91	3.89	5.96	35.45	5.95	0.95	0.91
			GPR	3.97	5.22	7.48	55.84	7.47	0.86	0.75
			EBT	2.62	3.47	5.22	27.23	5.22	0.96	0.92

10	13	50	FT	2.76	3.65	5.70	32.49	5.70	0.95	0.91
			GPR	2.49	3.33	4.81	23.14	4.81	0.96	0.93
			EBT	2.47	3.27	4.85	23.50	4.85	0.96	0.93

11	25	100	FT	2.24	3.00	5.14	26.41	5.14	0.97	0.94
			GPR	**2.00**	**2.68**	**4.38**	**19.19**	**4.38**	**0.98**	**0.95**
			EBT	2.05	2.72	4.39	19.22	4.38	0.98	0.95

L: level; FN: number of feature; FP: percentage of feature; FT: fine tree; GPR: Gaussian process regression; EBT: ensemble bagged tree.

**Table 11:** SBP prediction models for 16-second epoching.

Info				Performance evaluation criteria						
L	FN	FP	Model	MAPE	MAD	SE	MSE	RMSE	*R*	*R* ^2^
1	1	5	FT	3.18	4.25	5.86	34.29	5.86	0.94	0.88
			GPR	2.87	3.82	5.17	26.64	5.16	0.94	0.89
			EBT	2.94	3.92	5.39	29.05	5.39	0.94	0.88

2	3	10	FT	3.07	4.11	5.76	33.10	5.75	0.94	0.89
			GPR	2.78	3.72	5.48	30.00	5.48	0.94	0.89
			EBT	2.78	3.70	5.24	27.42	5.24	0.95	0.90

3	4	15	FT	3.07	4.11	5.75	33.06	5.75	0.94	0.89
			GPR	5.33	7.27	124.66	15514.79	124.56	0.94	0.89
			EBT	2.77	3.69	5.18	26.80	5.18	0.95	0.90

4	5	20	FT	3.07	4.11	5.75	33.06	5.75	0.94	0.89
			GPR	6.77	9.27	192.70	37072.41	192.54	0.94	0.89
			EBT	2.79	3.71	5.27	27.68	5.26	0.95	0.90

5	6	25	FT	2.92	3.91	5.73	32.83	5.73	0.95	0.90
			GPR	8.36	11.48	268.79	72126.37	268.56	0.94	0.89
			EBT	2.67	3.54	5.13	26.29	5.13	0.96	0.91

6	8	30	FT	2.87	3.83	5.72	32.71	5.72	0.95	0.91
			GPR	6.49	8.86	179.87	32299.68	179.72	0.95	0.89
			EBT	2.53	3.36	4.98	24.77	4.98	0.96	0.92

7	9	35	FT	2.87	3.83	5.72	32.72	5.72	0.95	0.91
			GPR	63.68	88.44	2946.64	8668294.47	2944.20	0.95	0.90
			EBT	2.56	3.40	4.98	24.74	4.97	0.96	0.92

8	10	40	FT	2.91	3.88	5.75	33.03	5.75	0.95	0.90
			GPR	3.25	4.35	22.40	500.78	22.38	0.95	0.90
			EBT	2.54	3.38	4.91	24.10	4.91	0.96	0.92

9	11	45	FT	2.90	3.87	5.75	32.97	5.74	0.95	0.90
			GPR	5.67	7.73	138.96	19278.64	138.85	0.95	0.90
			EBT	2.53	3.36	4.95	24.47	4.95	0.96	0.92

10	13	50	FT	2.45	3.30	5.12	26.19	5.12	0.96	0.93
			GPR	2.50	3.33	4.91	24.05	4.90	0.96	0.92
			EBT	2.27	3.02	4.57	20.88	4.57	0.97	0.94

11	25	100	FT	2.00	2.69	4.66	21.70	4.66	0.98	0.95
			GPR	**1.92**	**2.56**	**4.09**	**16.66**	**4.08**	**0.98**	**0.96**
			EBT	1.95	2.60	4.22	17.80	4.22	0.98	0.96

L: level; FN: number of feature; FP: percentage of feature; FT: fine tree; GPR: Gaussian process regression; EBT: ensemble bagged tree.

**Table 12:** SBP prediction models for 18-second epoching.

Info				Performance evaluation criteria						
L	FN	FP	Model	MAPE	MAD	SE	MSE	RMSE	*R*	*R* ^2^
1	1	5	FT	5.28	6.93	9.64	92.73	9.63	0.75	0.57
			GPR	4.74	6.21	8.20	67.10	8.19	0.81	0.66
			EBT	4.92	6.45	8.86	78.40	8.85	0.77	0.60

2	3	10	FT	4.01	5.30	7.89	62.06	7.88	0.88	0.77
			GPR	4.55	5.97	7.80	60.80	7.80	0.85	0.72
			EBT	3.83	5.00	7.24	52.29	7.23	0.89	0.80

3	4	15	FT	4.17	5.51	8.18	66.86	8.18	0.87	0.75
			GPR	3.83	5.05	7.04	49.43	7.03	0.89	0.79
			EBT	3.66	4.82	7.00	48.94	7.00	0.89	0.80

4	5	20	FT	4.17	5.51	8.18	66.86	8.18	0.87	0.75
			GPR	3.83	5.05	7.02	49.13	7.01	0.89	0.79
			EBT	3.73	4.90	7.08	50.05	7.07	0.89	0.79

5	6	25	FT	4.17	5.51	8.18	66.86	8.18	0.87	0.75
			GPR	3.83	5.06	7.02	49.13	7.01	0.89	0.79
			EBT	3.71	4.89	7.02	49.22	7.02	0.89	0.80

6	8	30	FT	3.72	4.93	7.59	57.58	7.59	0.89	0.79
			GPR	3.71	4.90	6.92	47.74	6.91	0.89	0.80
			EBT	3.30	4.33	6.38	40.59	6.37	0.92	0.84

7	9	35	FT	3.72	4.93	7.59	57.58	7.59	0.89	0.79
			GPR	3.70	4.87	6.91	47.66	6.90	0.90	0.80
			EBT	3.34	4.39	6.43	41.24	6.42	0.92	0.84

8	10	40	FT	3.70	4.91	7.58	57.35	7.57	0.89	0.80
			GPR	3.70	4.88	6.89	47.33	6.88	0.90	0.80
			EBT	3.34	4.39	6.40	40.90	6.39	0.92	0.84

9	11	45	FT	3.70	4.91	7.58	57.37	7.57	0.89	0.79
			GPR	3.70	4.89	6.89	47.40	6.88	0.90	0.81
			EBT	3.40	4.47	6.51	42.34	6.51	0.91	0.84

10	13	50	FT	2.76	3.69	5.67	32.10	5.67	0.96	0.92
			GPR	2.65	3.56	5.13	26.25	5.12	0.96	0.91
			EBT	2.57	3.41	5.03	25.24	5.02	0.96	0.92

11	25	100	FT	2.12	2.84	4.91	24.04	4.90	0.97	0.94
			GPR	**1.97**	**2.63**	**4.38**	**19.18**	**4.38**	**0.97**	**0.95**
			EBT	1.99	2.64	4.39	19.27	4.39	0.98	0.95

L: level; FN: number of feature; FP: percentage of feature; FT: fine tree; GPR: Gaussian process regression; EBT: ensemble bagged tree.

**Table 13:** SBP prediction models for 20-second epoching.

Info				Performance evaluation criteria						
L	FN	FP	Model	MAPE	MAD	SE	MSE	RMSE	*R*	*R* ^2^
1	1	5	FT	5.03	6.59	9.31	86.53	9.30	0.76	0.58
			GPR	4.71	6.14	8.31	68.84	8.30	0.80	0.64
			EBT	4.76	6.22	8.61	73.99	8.60	0.78	0.60

2	3	10	FT	4.20	5.54	8.22	67.46	8.21	0.86	0.73
			GPR	3.95	5.19	7.36	54.01	7.35	0.87	0.75
			EBT	3.72	4.87	7.22	52.08	7.22	0.88	0.78

3	4	15	FT	4.20	5.55	8.22	67.49	8.22	0.86	0.73
			GPR	3.97	5.21	7.37	54.21	7.36	0.87	0.75
			EBT	3.73	4.90	7.25	52.45	7.24	0.88	0.77

4	5	20	FT	4.20	5.55	8.22	67.49	8.22	0.86	0.73
			GPR	3.98	5.22	7.39	54.54	7.38	0.87	0.75
			EBT	3.74	4.90	7.29	53.09	7.29	0.88	0.78

5	6	25	FT	3.83	5.04	7.54	56.69	7.53	0.88	0.78
			GPR	3.82	5.02	7.25	52.40	7.24	0.88	0.77
			EBT	3.39	4.43	6.73	45.15	6.72	0.91	0.82

6	8	30	FT	3.73	4.90	7.66	58.48	7.65	0.88	0.78
			GPR	3.65	4.81	6.92	47.83	6.92	0.89	0.79
			EBT	3.28	4.29	6.55	42.87	6.55	0.91	0.83

7	9	35	FT	3.73	4.90	7.66	58.48	7.65	0.88	0.78
			GPR	3.66	4.82	6.91	47.72	6.91	0.89	0.79
			EBT	3.36	4.39	6.72	45.04	6.71	0.91	0.82

8	10	40	FT	3.72	4.90	7.67	58.74	7.66	0.88	0.78
			GPR	3.65	4.80	6.90	47.51	6.89	0.89	0.79
			EBT	3.29	4.31	6.52	42.39	6.51	0.91	0.83

9	11	45	FT	3.72	4.90	7.67	58.75	7.66	0.88	0.78
			GPR	3.65	4.80	6.90	47.54	6.90	0.89	0.79
			EBT	3.32	4.35	6.62	43.70	6.61	0.91	0.83

10	13	50	FT	2.39	3.23	5.11	26.08	5.11	0.96	0.93
			GPR	2.44	3.26	4.80	23.00	4.80	0.96	0.92
			EBT	2.28	3.02	4.70	22.05	4.70	0.97	0.93

11	25	100	FT	2.17	2.89	5.15	26.43	5.14	0.97	0.94
			GPR	**1.96**	**2.62**	**4.13**	**16.98**	**4.12**	**0.98**	**0.96**
			EBT	1.96	2.60	4.29	18.41	4.29	0.98	0.95

L: level; FN: number of feature; FP: percentage of feature; FT: fine tree; GPR: Gaussian process regression; EBT: ensemble bagged tree.

**Table 14:** DBP prediction models for 2-second epoching.

Info				Performance evaluation criteria						
L	FN	FP	Model	MAPE	MAD	SE	MSE	RMSE	*R*	*R* ^2^
1	1	5	FT	8.43	6.18	8.32	69.21	8.32	0.62	0.39
			GPR	7.31	5.32	7.10	50.40	7.10	0.66	0.44
			EBT	7.69	5.62	7.52	56.61	7.52	0.64	0.41

2	3	10	FT	6.47	4.80	7.25	52.54	7.25	0.79	0.62
			GPR	6.99	5.10	6.88	47.33	6.88	0.73	0.53
			EBT	5.53	4.06	6.03	36.37	6.03	0.83	0.69

3	4	15	FT	6.16	4.56	7.00	48.97	7.00	0.81	0.66
			GPR	5.98	4.38	6.21	38.52	6.21	0.82	0.67
			EBT	5.22	3.85	5.77	33.30	5.77	0.85	0.73

4	5	20	FT	6.16	4.56	7.00	48.97	7.00	0.81	0.66
			GPR	5.96	4.36	6.19	38.34	6.19	0.82	0.67
			EBT	5.25	3.86	5.80	33.59	5.80	0.85	0.73

5	6	25	FT	6.17	4.56	7.02	49.30	7.02	0.81	0.66
			GPR	5.89	4.31	6.16	37.93	6.16	0.82	0.68
			EBT	5.25	3.86	5.78	33.40	5.78	0.85	0.73

6	8	30	FT	6.19	4.57	7.04	49.48	7.03	0.81	0.66
			GPR	5.99	4.39	6.21	38.56	6.21	0.81	0.66
			EBT	5.26	3.86	5.81	33.69	5.80	0.85	0.73

7	9	35	FT	5.65	4.17	6.55	42.94	6.55	0.85	0.72
			GPR	5.58	4.09	5.95	35.36	5.95	0.84	0.70
			EBT	5.01	3.68	5.57	31.07	5.57	0.87	0.76

8	10	40	FT	5.26	3.90	6.20	38.44	6.20	0.87	0.76
			GPR	5.07	3.73	5.49	30.13	5.49	0.88	0.77
			EBT	4.58	3.38	5.20	27.08	5.20	0.90	0.81

9	11	45	FT	5.26	3.89	6.20	38.39	6.20	0.87	0.76
			GPR	4.93	3.63	5.39	29.02	5.39	0.88	0.78
			EBT	4.60	3.39	5.20	27.03	5.20	0.90	0.81

10	13	50	FT	4.15	3.11	5.20	27.06	5.20	0.95	0.90
			GPR	3.65	2.68	4.31	18.57	4.31	0.96	0.92
			EBT	3.50	2.58	4.26	18.16	4.26	0.96	0.92

11	25	100	FT	4.06	3.03	5.23	27.33	5.23	0.95	0.91
			GPR	3.56	2.61	4.21	17.70	4.21	0.96	0.92
			EBT	**3.31**	**2.43**	**4.06**	**16.52**	**4.06**	**0.97**	**0.93**

L: level; FN: number of feature; FP: percentage of feature; FT: fine tree; GPR: Gaussian process regression; EBT: ensemble bagged tree.

**Table 15:** DBP prediction models for 4-second epoching.

Info				Performance evaluation criteria						
L	FN	FP	Model	MAPE	MAD	SE	MSE	RMSE	*R*	*R* ^2^
1	1	5	FT	7.92	5.75	7.89	62.24	7.89	0.63	0.40
			GPR	7.10	5.11	6.87	47.21	6.87	0.65	0.43
			EBT	7.40	5.34	7.27	52.86	7.27	0.64	0.41

2	3	10	FT	4.87	3.53	5.57	31.06	5.57	0.92	0.85
			GPR	5.00	3.56	5.34	28.54	5.34	0.90	0.82
			EBT	4.11	2.93	4.71	22.13	4.70	0.94	0.88

3	4	15	FT	4.69	3.39	5.44	29.59	5.44	0.93	0.86
			GPR	4.21	3.01	4.77	22.72	4.77	0.93	0.86
			EBT	3.97	2.83	4.55	20.67	4.55	0.94	0.89

4	5	20	FT	4.69	3.39	5.44	29.59	5.44	0.93	0.86
			GPR	4.17	2.98	4.74	22.41	4.73	0.93	0.86
			EBT	3.97	2.83	4.56	20.81	4.56	0.94	0.88

5	6	25	FT	4.68	3.37	5.47	29.93	5.47	0.93	0.86
			GPR	4.21	3.01	4.77	22.71	4.77	0.93	0.86
			EBT	3.98	2.84	4.57	20.91	4.57	0.94	0.88

6	8	30	FT	4.72	3.40	5.49	30.11	5.49	0.93	0.86
			GPR	4.20	3.00	4.75	22.59	4.75	0.93	0.86
			EBT	4.01	2.86	4.60	21.13	4.60	0.94	0.88

7	9	35	FT	4.60	3.34	5.39	29.04	5.39	0.93	0.86
			GPR	4.02	2.86	4.61	21.21	4.61	0.94	0.88
			EBT	3.92	2.79	4.53	20.53	4.53	0.94	0.89

8	10	40	FT	4.44	3.20	5.24	27.42	5.24	0.93	0.87
			GPR	3.84	2.73	4.45	19.83	4.45	0.94	0.89
			EBT	3.74	2.66	4.39	19.28	4.39	0.95	0.90

9	11	45	FT	4.44	3.20	5.24	27.42	5.24	0.93	0.87
			GPR	3.86	2.75	4.46	19.92	4.46	0.94	0.89
			EBT	3.74	2.67	4.40	19.32	4.40	0.95	0.90

10	13	50	FT	3.97	2.84	4.76	22.60	4.75	0.96	0.91
			GPR	3.42	2.42	3.99	15.92	3.99	0.96	0.93
			EBT	3.39	2.40	4.04	16.32	4.04	0.96	0.93

11	25	100	FT	3.76	2.68	4.74	22.41	4.73	0.96	0.92
			GPR	3.28	2.31	3.89	15.15	3.89	0.97	0.94
			EBT	**3.17**	**2.24**	**3.85**	**14.82**	**3.85**	**0.97**	**0.94**

L: level; FN: number of feature; FP: percentage of feature; FT: fine tree; GPR: Gaussian process regression; EBT: ensemble bagged tree.

**Table 16:** DBP prediction models for 6-second epoching.

Info				Performance evaluation criteria						
L	FN	FP	Model	MAPE	MAD	SE	MSE	RMSE	*R*	*R* ^2^
1	1	5	FT	7.74	5.50	7.71	59.44	7.71	0.65	0.42
			GPR	6.80	4.79	6.64	44.00	6.63	0.71	0.50
			EBT	7.18	5.07	7.06	49.84	7.06	0.67	0.45

2	3	10	FT	6.40	4.52	6.87	47.23	6.87	0.79	0.62
			GPR	6.94	4.89	6.67	44.52	6.67	0.70	0.49
			EBT	5.77	4.01	5.89	34.73	5.89	0.83	0.68

3	4	15	FT	6.40	4.51	6.87	47.11	6.86	0.79	0.62
			GPR	6.92	4.87	6.67	44.41	6.66	0.70	0.49
			EBT	5.71	3.99	5.90	34.74	5.89	0.83	0.68

4	5	20	FT	6.40	4.51	6.87	47.11	6.86	0.79	0.62
			GPR	6.89	4.85	6.66	44.34	6.66	0.71	0.51
			EBT	5.73	3.99	5.91	34.85	5.90	0.82	0.68

5	6	25	FT	6.41	4.57	7.07	49.97	7.07	0.79	0.62
			GPR	6.24	4.37	6.28	39.43	6.28	0.78	0.61
			EBT	5.57	3.90	5.85	34.23	5.85	0.83	0.70

6	8	30	FT	6.38	4.57	7.02	49.27	7.02	0.79	0.62
			GPR	6.15	4.31	6.23	38.81	6.23	0.78	0.61
			EBT	5.54	3.88	5.82	33.85	5.82	0.84	0.70

7	9	35	FT	6.39	4.53	6.99	48.88	6.99	0.80	0.63
			GPR	6.16	4.31	6.22	38.65	6.22	0.78	0.61
			EBT	5.53	3.88	5.82	33.88	5.82	0.84	0.70

8	10	40	FT	6.40	4.55	7.00	48.94	7.00	0.79	0.62
			GPR	6.14	4.30	6.22	38.65	6.22	0.78	0.61
			EBT	5.56	3.89	5.85	34.24	5.85	0.83	0.69

9	11	45	FT	5.87	4.14	6.61	43.68	6.61	0.83	0.70
			GPR	5.94	4.14	6.02	36.22	6.02	0.81	0.65
			EBT	5.27	3.67	5.61	31.45	5.61	0.86	0.73

10	13	50	FT	3.96	2.75	4.70	22.04	4.69	0.95	0.91
			GPR	3.60	2.46	4.11	16.85	4.10	0.96	0.92
			EBT	3.46	2.38	4.04	16.35	4.04	0.96	0.92

11	25	100	FT	3.53	2.52	4.43	19.62	4.43	0.96	0.92
			GPR	3.32	2.27	3.87	15.00	3.87	0.97	0.94
			EBT	**3.14**	**2.15**	**3.79**	**14.34**	**3.79**	**0.97**	**0.94**

L: level; FN: number of feature; FP: percentage of feature; FT: fine tree; GPR: Gaussian process regression; EBT: ensemble bagged tree.

**Table 17:** DBP prediction models for 8-second epoching.

Info				Performance evaluation criteria						
L	FN	FP	Model	MAPE	MAD	SE	MSE	RMSE	*R*	*R* ^2^
1	1	5	FT	7.05	5.13	7.26	52.72	7.26	0.67	0.45
			GPR	6.41	4.59	6.25	39.05	6.25	0.73	0.53
			EBT	6.73	4.76	6.68	44.60	6.68	0.71	0.50

2	3	10	FT	5.55	3.89	6.03	36.30	6.03	0.85	0.73
			GPR	6.43	4.44	6.24	38.86	6.23	0.77	0.59
			EBT	5.60	3.85	5.70	32.41	5.69	0.84	0.71

3	4	15	FT	5.55	3.89	6.03	36.33	6.03	0.85	0.73
			GPR	6.43	4.44	6.25	39.00	6.25	0.77	0.59
			EBT	5.57	3.84	5.71	32.56	5.71	0.84	0.70

4	5	20	FT	5.55	3.89	6.03	36.33	6.03	0.85	0.73
			GPR	6.47	4.47	6.26	39.10	6.25	0.76	0.58
			EBT	5.68	3.92	5.80	33.57	5.79	0.83	0.69

5	6	25	FT	5.80	4.02	6.28	39.35	6.27	0.83	0.69
			GPR	6.45	4.45	6.26	39.15	6.26	0.77	0.59
			EBT	5.27	3.61	5.46	29.75	5.45	0.86	0.74

6	8	30	FT	5.95	4.09	6.39	40.82	6.39	0.83	0.68
			GPR	5.89	4.04	5.92	35.04	5.92	0.81	0.66
			EBT	5.10	3.47	5.33	28.33	5.32	0.87	0.76

7	9	35	FT	5.95	4.09	6.39	40.82	6.39	0.83	0.68
			GPR	5.83	4.00	5.87	34.40	5.87	0.82	0.67
			EBT	5.13	3.49	5.36	28.73	5.36	0.87	0.76

8	10	40	FT	5.96	4.10	6.46	41.71	6.46	0.83	0.68
			GPR	5.76	3.96	5.83	33.97	5.83	0.82	0.67
			EBT	5.10	3.45	5.36	28.68	5.36	0.87	0.76

9	11	45	FT	5.98	4.11	6.49	42.11	6.49	0.82	0.68
			GPR	5.78	3.97	5.84	34.03	5.83	0.82	0.68
			EBT	5.14	3.49	5.38	28.88	5.37	0.87	0.76

10	13	50	FT	5.50	3.87	6.15	37.73	6.14	0.85	0.72
			GPR	5.60	3.82	5.67	32.07	5.66	0.84	0.70
			EBT	4.93	3.36	5.23	27.32	5.23	0.88	0.78

11	25	100	FT	3.31	2.35	4.23	17.90	4.23	0.96	0.93
			GPR	3.23	2.11	3.59	12.86	3.59	0.97	0.94
			EBT	**3.11**	**2.04**	**3.63**	**13.19**	**3.63**	**0.97**	**0.95**

L: level; FN: number of feature; FP: percentage of feature; FT: fine tree; GPR: Gaussian process regression; EBT: ensemble bagged tree.

**Table 18:** DBP prediction models for 10-second epoching.

Info				Performance evaluation criteria						
L	FN	FP	Model	MAPE	MAD	SE	MSE	RMSE	*R*	*R* ^2^
1	1	5	FT	6.56	4.86	6.93	48.00	6.93	0.71	0.50
			GPR	5.99	4.42	6.05	36.51	6.04	0.75	0.57
			EBT	6.14	4.52	6.35	40.26	6.35	0.74	0.54

2	3	10	FT	6.04	4.47	6.75	45.55	6.75	0.77	0.59
			GPR	5.85	4.32	5.98	35.71	5.98	0.76	0.58
			EBT	5.51	4.03	5.93	35.13	5.93	0.81	0.65

3	4	15	FT	6.04	4.47	6.75	45.55	6.75	0.77	0.59
			GPR	5.86	4.32	5.98	35.76	5.98	0.76	0.58
			EBT	5.48	4.02	5.92	35.04	5.92	0.81	0.65

4	5	20	FT	6.03	4.46	6.80	46.14	6.79	0.78	0.60
			GPR	5.66	4.15	5.94	35.19	5.93	0.79	0.62
			EBT	5.36	3.92	5.86	34.32	5.86	0.82	0.67

5	6	25	FT	5.34	3.96	6.08	36.90	6.07	0.83	0.69
			GPR	5.68	4.15	5.95	35.36	5.95	0.79	0.62
			EBT	4.89	3.58	5.42	29.31	5.41	0.86	0.74

6	8	30	FT	5.62	4.11	6.51	42.36	6.51	0.82	0.67
			GPR	5.20	3.81	5.63	31.65	5.63	0.83	0.69
			EBT	4.73	3.44	5.36	28.74	5.36	0.87	0.75

7	9	35	FT	5.59	4.08	6.48	41.89	6.47	0.82	0.68
			GPR	5.20	3.80	5.64	31.73	5.63	0.83	0.69
			EBT	4.75	3.46	5.40	29.13	5.40	0.86	0.75

8	10	40	FT	5.65	4.13	6.50	42.24	6.50	0.82	0.67
			GPR	5.21	3.81	5.61	31.48	5.61	0.83	0.68
			EBT	4.74	3.45	5.38	28.95	5.38	0.87	0.75

9	11	45	FT	5.60	4.09	6.48	41.90	6.47	0.82	0.68
			GPR	5.18	3.80	5.60	31.32	5.60	0.83	0.69
			EBT	4.75	3.45	5.39	29.03	5.39	0.87	0.75

10	13	50	FT	3.66	2.73	4.58	21.00	4.58	0.95	0.90
			GPR	3.27	2.40	3.84	14.71	3.84	0.96	0.92
			EBT	3.23	2.36	3.87	14.94	3.86	0.96	0.92

11	25	100	FT	3.05	2.30	4.16	17.32	4.16	0.96	0.93
			GPR	2.85	2.08	3.53	12.46	3.53	0.97	0.94
			EBT	**2.69**	**1.96**	**3.42**	**11.67**	**3.42**	**0.97**	**0.95**

L: level; FN: number of feature; FP: percentage of feature; FT: fine tree; GPR: Gaussian process regression; EBT: ensemble bagged tree.

**Table 19:** DBP prediction models for 12-second epoching.

Info				Performance evaluation criteria						
L	FN	FP	Model	MAPE	MAD	SE	MSE	RMSE	*R*	*R* ^2^
1	1	5	FT	6.68	4.75	6.85	46.83	6.84	0.71	0.50
			GPR	5.97	4.20	5.89	34.62	5.88	0.78	0.60
			EBT	6.19	4.37	6.22	38.69	6.22	0.74	0.55

2	3	10	FT	5.83	4.12	6.21	38.47	6.20	0.81	0.66
			GPR	5.77	4.07	5.73	32.84	5.73	0.79	0.63
			EBT	5.38	3.69	5.54	30.68	5.54	0.84	0.71

3	4	15	FT	5.83	4.12	6.21	38.47	6.20	0.81	0.66
			GPR	5.77	4.07	5.74	32.88	5.73	0.79	0.63
			EBT	5.28	3.64	5.50	30.19	5.49	0.84	0.71

4	5	20	FT	5.79	4.09	6.24	38.90	6.24	0.83	0.68
			GPR	5.52	3.86	5.65	31.93	5.65	0.81	0.66
			EBT	5.33	3.63	5.52	30.40	5.51	0.85	0.71

5	6	25	FT	5.15	3.62	5.71	32.59	5.71	0.88	0.77
			GPR	4.72	3.28	5.07	25.63	5.06	0.88	0.77
			EBT	4.78	3.23	4.99	24.88	4.99	0.89	0.80

6	8	30	FT	4.84	3.39	5.43	29.42	5.42	0.89	0.79
			GPR	4.54	3.17	4.92	24.16	4.92	0.89	0.79
			EBT	4.35	2.91	4.65	21.57	4.64	0.92	0.84

7	9	35	FT	4.84	3.39	5.43	29.42	5.42	0.89	0.79
			GPR	4.48	3.14	4.86	23.58	4.86	0.89	0.79
			EBT	4.39	2.93	4.72	22.22	4.71	0.91	0.84

8	10	40	FT	4.85	3.39	5.44	29.55	5.44	0.89	0.79
			GPR	4.48	3.14	4.85	23.53	4.85	0.89	0.79
			EBT	4.40	2.94	4.72	22.21	4.71	0.91	0.83

9	11	45	FT	4.81	3.37	5.44	29.53	5.43	0.89	0.80
			GPR	4.48	3.13	4.85	23.50	4.85	0.89	0.79
			EBT	4.40	2.95	4.72	22.21	4.71	0.91	0.83

10	13	50	FT	3.91	2.71	4.49	20.12	4.49	0.95	0.90
			GPR	3.60	2.48	3.99	15.91	3.99	0.95	0.91
			EBT	3.57	2.34	3.95	15.56	3.95	0.96	0.92

11	25	100	FT	3.15	2.17	4.01	16.09	4.01	0.97	0.94
			GPR	**2.88**	**1.99**	**3.49**	**12.18**	**3.49**	**0.97**	**0.95**
			EBT	3.01	1.95	3.52	12.35	3.51	0.97	0.95

L: level; FN: number of feature; FP: percentage of feature; FT: fine tree; GPR: Gaussian process regression; EBT: ensemble bagged tree.

**Table 20:** DBP prediction models for 14-second epoching.

Info				Performance evaluation criteria						
L	FN	FP	Model	MAPE	MAD	SE	MSE	RMSE	*R*	*R* ^2^
1	1	5	FT	4.62	3.18	4.55	20.68	4.55	0.92	0.84
			GPR	3.98	2.68	3.97	15.75	3.97	0.94	0.88
			EBT	4.28	2.92	4.22	17.82	4.22	0.93	0.86

2	3	10	FT	4.18	2.83	4.29	18.36	4.29	0.94	0.89
			GPR	4.16	2.83	8.41	70.58	8.40	0.94	0.88
			EBT	4.24	2.64	4.44	19.69	4.44	0.94	0.88

3	4	15	FT	4.18	2.83	4.29	18.36	4.29	0.94	0.89
			GPR	4.24	2.90	9.98	99.45	9.97	0.94	0.88
			EBT	4.04	2.57	4.13	17.04	4.13	0.95	0.90

4	5	20	FT	4.25	2.92	4.40	19.29	4.39	0.94	0.89
			GPR	9.65	7.18	174.80	30511.96	174.68	0.95	0.89
			EBT	4.07	2.57	4.17	17.37	4.17	0.95	0.90

5	6	25	FT	4.10	2.77	4.41	19.42	4.41	0.95	0.91
			GPR	4.85	3.31	23.40	546.56	23.38	0.95	0.90
			EBT	3.83	2.41	4.04	16.32	4.04	0.96	0.91

6	8	30	FT	4.18	2.64	4.55	20.69	4.55	0.95	0.91
			GPR	4.45	3.28	28.94	836.05	28.91	0.94	0.89
			EBT	3.77	2.35	3.96	15.65	3.96	0.96	0.92

7	9	35	FT	4.18	2.64	4.55	20.69	4.55	0.95	0.91
			GPR	4.51	2.86	9.87	97.34	9.87	0.95	0.90
			EBT	3.87	2.39	4.06	16.44	4.05	0.96	0.92

8	10	40	FT	4.18	2.64	4.55	20.71	4.55	0.95	0.91
			GPR	5.30	3.38	5.29	27.93	5.28	0.87	0.75
			EBT	3.80	2.34	3.98	15.85	3.98	0.96	0.92

9	11	45	FT	4.16	2.62	4.53	20.53	4.53	0.95	0.91
			GPR	5.19	3.83	40.68	1652.57	40.65	0.95	0.90
			EBT	3.88	2.37	4.06	16.49	4.06	0.96	0.92

10	13	50	FT	3.75	2.51	4.18	17.43	4.17	0.95	0.91
			GPR	3.60	2.26	3.77	14.22	3.77	0.96	0.92
			EBT	3.65	2.22	3.84	14.72	3.84	0.96	0.93

11	25	100	FT	3.18	2.07	3.82	14.57	3.82	0.97	0.94
			GPR	3.37	1.97	3.66	13.40	3.66	0.97	0.95
			EBT	**3.28**	**1.87**	**3.64**	**13.25**	**3.64**	**0.98**	**0.95**

L: level; FN: number of feature; FP: percentage of feature; FT: fine tree; GPR: Gaussian process regression; EBT: ensemble bagged tree.

**Table 21:** DBP prediction models for 16-second epoching.

Info				Performance evaluation criteria						
L	FN	FP	Model	MAPE	MAD	SE	MSE	RMSE	*R*	*R* ^2^
1	1	5	FT	3.71	2.81	4.17	17.33	4.16	0.94	0.88
			GPR	3.33	2.50	3.72	13.84	3.72	0.94	0.89
			EBT	3.46	2.61	3.88	15.02	3.88	0.94	0.88

2	3	10	FT	3.62	2.76	4.04	16.32	4.04	0.95	0.89
			GPR	3.87	2.96	19.45	377.68	19.43	0.94	0.89
			EBT	3.34	2.48	3.86	14.86	3.85	0.95	0.90

3	4	15	FT	3.62	2.76	4.04	16.32	4.04	0.95	0.89
			GPR	5.93	4.62	76.65	5865.87	76.59	0.94	0.89
			EBT	3.34	2.50	3.79	14.34	3.79	0.95	0.90

4	5	20	FT	3.62	2.76	4.04	16.32	4.04	0.95	0.89
			GPR	7.76	6.09	127.74	16289.21	127.63	0.94	0.89
			EBT	3.35	2.50	3.87	14.93	3.86	0.95	0.90

5	6	25	FT	3.31	2.52	4.03	16.23	4.03	0.95	0.91
			GPR	6.20	4.84	84.13	7066.21	84.06	0.94	0.89
			EBT	3.19	2.36	3.76	14.09	3.75	0.96	0.91

6	8	30	FT	3.46	2.62	4.13	17.06	4.13	0.95	0.90
			GPR	21.04	16.78	499.07	248655.06	498.65	0.95	0.90
			EBT	3.04	2.26	3.59	12.87	3.59	0.96	0.92

7	9	35	FT	3.45	2.62	4.13	17.03	4.13	0.95	0.90
			GPR	20.87	16.64	493.67	243303.01	493.26	0.95	0.90
			EBT	3.08	2.29	3.69	13.56	3.68	0.96	0.92

8	10	40	FT	3.37	2.55	4.07	16.55	4.07	0.95	0.90
			GPR	5.70	4.41	67.87	4599.29	67.82	0.95	0.89
			EBT	3.06	2.28	3.66	13.41	3.66	0.96	0.92

9	11	45	FT	3.37	2.55	4.07	16.55	4.07	0.95	0.90
			GPR	4.36	3.24	4.94	24.34	4.93	0.88	0.78
			EBT	3.10	2.30	3.72	13.80	3.72	0.96	0.92

10	13	50	FT	3.06	2.32	3.74	13.95	3.73	0.96	0.92
			GPR	3.01	2.26	3.59	12.89	3.59	0.96	0.92
			EBT	2.85	2.11	3.51	12.30	3.51	0.97	0.93

11	25	100	FT	2.61	1.99	3.71	13.73	3.71	0.97	0.95
			GPR	**2.44**	**1.83**	**3.11**	**9.64**	**3.10**	**0.98**	**0.95**
			EBT	2.44	1.81	3.23	10.42	3.23	0.98	0.95

L: level; FN: number of feature; FP: percentage of feature; FT: fine tree; GPR: Gaussian process regression; EBT: ensemble bagged tree.

**Table 22:** DBP prediction models for 18-second epoching.

Info				Performance evaluation criteria						
L	FN	FP	Model	MAPE	MAD	SE	MSE	RMSE	*R*	*R* ^2^
1	1	5	FT	5.86	4.37	6.31	39.75	6.30	0.76	0.57
			GPR	5.21	3.87	5.41	29.17	5.40	0.82	0.67
			EBT	5.44	4.04	5.76	33.14	5.76	0.78	0.61

2	3	10	FT	4.65	3.49	5.31	28.19	5.31	0.87	0.76
			GPR	5.00	3.72	5.16	26.57	5.15	0.85	0.72
			EBT	4.29	3.15	4.85	23.52	4.85	0.89	0.80

3	4	15	FT	4.75	3.56	5.50	30.17	5.49	0.86	0.75
			GPR	4.27	3.18	4.68	21.90	4.68	0.89	0.79
			EBT	4.15	3.08	4.69	21.98	4.69	0.89	0.80

4	5	20	FT	4.75	3.56	5.50	30.17	5.49	0.86	0.75
			GPR	4.26	3.18	4.67	21.75	4.66	0.89	0.79
			EBT	4.19	3.11	4.77	22.67	4.76	0.89	0.79

5	6	25	FT	4.75	3.56	5.50	30.17	5.49	0.86	0.75
			GPR	4.25	3.17	4.65	21.60	4.65	0.89	0.79
			EBT	4.16	3.09	4.72	22.23	4.71	0.89	0.80

6	8	30	FT	4.41	3.32	5.27	27.74	5.27	0.89	0.79
			GPR	4.14	3.09	4.62	21.32	4.62	0.89	0.80
			EBT	3.78	2.80	4.35	18.93	4.35	0.91	0.84

7	9	35	FT	4.41	3.32	5.27	27.74	5.27	0.89	0.79
			GPR	4.13	3.08	4.60	21.15	4.60	0.90	0.80
			EBT	3.78	2.79	4.36	19.00	4.36	0.92	0.84

8	10	40	FT	4.41	3.32	5.27	27.74	5.27	0.89	0.79
			GPR	4.13	3.08	4.59	21.06	4.59	0.90	0.81
			EBT	3.78	2.80	4.35	18.87	4.34	0.91	0.84

9	11	45	FT	4.41	3.32	5.27	27.73	5.27	0.89	0.79
			GPR	4.14	3.09	4.60	21.09	4.59	0.90	0.81
			EBT	3.81	2.82	4.38	19.19	4.38	0.92	0.84

10	13	50	FT	3.21	2.43	3.99	15.89	3.99	0.96	0.91
			GPR	3.05	2.30	3.53	12.42	3.52	0.96	0.91
			EBT	2.98	2.20	3.54	12.48	3.53	0.96	0.93

11	25	100	FT	2.58	1.95	3.63	13.17	3.63	0.97	0.94
			GPR	2.53	1.89	3.39	11.48	3.39	0.97	0.94
			EBT	**2.49**	**1.83**	**3.24**	**10.45**	**3.23**	**0.97**	**0.95**

L: level; FN: number of feature; FP: percentage of feature; FT: fine tree; GPR: Gaussian process regression; EBT: ensemble bagged tree.

**Table 23:** DBP prediction models for 20-second epoching.

Info				Performance evaluation criteria						
L	FN	FP	Model	MAPE	MAD	SE	MSE	RMSE	*R*	*R* ^2^
1	1	5	FT	5.58	4.16	6.09	36.96	6.08	0.77	0.59
			GPR	5.21	3.85	5.48	29.96	5.47	0.80	0.63
			EBT	5.25	3.91	5.65	31.89	5.65	0.78	0.61

2	3	10	FT	4.66	3.48	5.35	28.52	5.34	0.86	0.75
			GPR	4.39	3.26	4.90	23.97	4.90	0.87	0.76
			EBT	4.26	3.14	4.92	24.16	4.92	0.88	0.77

3	4	15	FT	4.65	3.47	5.34	28.48	5.34	0.86	0.75
			GPR	4.41	3.28	4.91	24.06	4.91	0.87	0.75
			EBT	4.20	3.11	4.89	23.84	4.88	0.88	0.77

4	5	20	FT	4.65	3.47	5.34	28.48	5.34	0.86	0.75
			GPR	4.29	3.18	4.89	23.83	4.88	0.88	0.77
			EBT	4.23	3.13	4.91	24.10	4.91	0.88	0.77

5	6	25	FT	4.19	3.14	4.86	23.54	4.85	0.89	0.79
			GPR	4.39	3.26	4.93	24.26	4.93	0.87	0.76
			EBT	3.87	2.84	4.58	20.89	4.57	0.91	0.82

6	8	30	FT	4.24	3.15	5.12	26.12	5.11	0.88	0.78
			GPR	4.05	3.02	4.64	21.47	4.63	0.89	0.79
			EBT	3.75	2.77	4.45	19.80	4.45	0.91	0.83

7	9	35	FT	4.24	3.15	5.12	26.12	5.11	0.88	0.78
			GPR	4.04	3.00	4.63	21.40	4.63	0.89	0.79
			EBT	3.83	2.83	4.53	20.49	4.53	0.91	0.82

8	10	40	FT	4.26	3.17	5.15	26.43	5.14	0.88	0.78
			GPR	4.04	3.00	4.62	21.33	4.62	0.89	0.79
			EBT	3.76	2.77	4.51	20.27	4.50	0.91	0.83

9	11	45	FT	4.25	3.15	5.14	26.33	5.13	0.88	0.78
			GPR	4.06	3.02	4.63	21.44	4.63	0.89	0.79
			EBT	3.78	2.79	4.49	20.14	4.49	0.91	0.83

10	13	50	FT	2.90	2.19	3.67	13.45	3.67	0.96	0.93
			GPR	2.86	2.13	3.41	11.59	3.40	0.96	0.93
			EBT	2.76	2.04	3.43	11.76	3.43	0.96	0.93

11	25	100	FT	2.72	2.02	3.77	14.17	3.76	0.97	0.94
			GPR	**2.49**	**1.85**	**3.14**	**9.82**	**3.13**	**0.97**	**0.95**
			EBT	2.37	1.75	3.17	10.04	3.17	0.97	0.95

L: level; FN: number of feature; FP: percentage of feature; FT: fine tree; GPR: Gaussian process regression; EBT: ensemble bagged tree.

**Table 24:** Performance chart of the best algorithms for the entire epoching process.

Info				Performance evaluation criteria						
ES	BP	FN	Model	MAPE	MAD	SE	MSE	RMSE	*R*	*R* ^2^
2	SBP	11	EBT	2.58	3.37	5.05	25.48	5.05	0.97	0.93
	DBP	11	EBT	3.31	2.43	4.06	16.52	4.06	0.97	0.93
4	SBP	11	EBT	2.34	3.09	4.86	23.62	4.86	0.97	0.94
	DBP	11	EBT	3.17	2.24	3.85	14.82	3.85	0.97	0.94
6	SBP	11	EBT	2.27	3.00	4.83	23.31	4.83	0.97	0.94
	DBP	11	EBT	3.14	2.15	3.79	14.34	3.79	0.97	0.94
8	SBP	11	GPR	2.20	2.91	4.50	20.28	4.50	0.97	0.95
	DBP	11	EBT	3.11	2.04	3.63	13.19	3.63	0.97	0.95
10	SBP	11	EBT	2.08	2.75	4.37	19.11	4.37	0.97	0.95
	DBP	11	EBT	2.69	1.96	3.42	11.67	3.42	0.97	0.95
12	SBP	11	GPR	2.04	2.73	4.39	19.25	4.39	0.98	0.95
	DBP	11	GPR	2.88	1.99	3.49	12.18	3.49	0.97	0.95
14	SBP	11	GPR	2.00	2.68	4.38	19.19	4.38	0.98	0.95
	DBP	11	EBT	3.28	1.87	3.64	13.25	3.64	0.98	0.95
16	SBP	11	GPR	**1.92**	**2.56**	**4.09**	**16.66**	**4.08**	**0.98**	**0.96**
	DBP	11	GPR	**2.44**	**1.83**	**3.11**	**9.64**	**3.10**	**0.98**	**0.95**
18	SBP	11	GPR	1.97	2.63	4.38	19.18	4.38	0.97	0.95
	DBP	11	EBT	2.49	1.83	3.24	10.45	3.23	0.97	0.95
20	SBP	11	GPR	1.96	2.62	4.13	16.98	4.12	0.98	0.96
	DBP	11	EBT	2.37	1.75	3.17	10.04	3.17	0.97	0.95

ES: epoch second; FN: number of feature; BP: blood pressure; SBP: systolic blood pressure; DBP: diastolic blood pressure; EBT: ensemble bagged tree; GPR: Gaussian process regression.

**Table 25:** Literature comparison.

Nu	Ref	Year	Model methods				Diastolic blood pressure performances						Systolic blood pressure performances [b]						
			Signal	Features	Method	MAE	MAPE	MAD	MSE	RMSE	*R*	*R* ^2^	MAE	MAPE	MAD	MSE	RMSE	=*R*	*R* ^2^
1	[33]	2019	PPT-PIR	SSR-CHC	MARS		3.630								7.830				
2	[29]	2020	Oscillometric waveforms	Graphical features	WkNN	11.032			200.531	14.161	0.423	0.179	3.520			41.998	6.480	0.948	0.899
3	[31]	2020	Auscultatory and oscillometric waveforms	Time domain	GMM-HMM	2.900							-0.9						
4	[34]	2020	PPG-ECG	Chaotic, time, and frequency domain	RNN				1.730	1.240	0.854	0.730				1.210	0.780	0.849	0.720
5	[30]	2020	Oscillometric waveforms	Chaotic, time, and frequency domain	GPR	4.271	0.288		28.843	5.371	0.891	0.794	3.636	0.114		23.845	4.883	0.962	0.925
6	[27]	2020	PPG-ECG	Time domain	RF	5.48				6.000	0.840	0.706	9.000				13.830	0.850	0.723
7	[32]	2020	Speech	Vowels	CNN-R					0.350							0.236		
8	[28]	2020	PPG	PPG segment series	CNN-LSTM	3.97					0.950	0.903		0.670				0.950	0.903
9	[26]	2021	Peripheral signals	Hibrit	MLR					3.000	0.970	0.941					3.000	0.970	0.941
10	[20]	2021	PPG	Multitype feature	MTFF-ANN	3.36							5.590						
11			Proposed model ECG 2-second	Time domain	EBT		3.310	2.430	16.520	4.060	0.970	0.930		2.580	0.370	25.480	5.050	0.970	0.930
12			Proposed model-ECG 14-second	Time domain	GPR/EBT		3.280	1.870	13.250	3.340	0.980	0.950		2.000	2.680	19.190	4.380	0.980	0.950
13			Proposed model-ECG 16-second	Time domain	GPR		2.440	1.830	9.640	3.100	0.980	0.950		1.920	2.560	16.660	4.080	0.980	0.960

CHC: current heart cycle; CNN-R: convolutional neural networks-regression; EBT: ensemble bagged tree; ECG: electrocardiography; GMM-HMM: Gaussian mixture models and hidden Markov; GPR: Gaussian process regression; LSTM: long-short-term memory; MAD: mean absolute difference; MAE: mean absolute error; MAPE: mean absolute percentage error; MAPE: mean absolute percentage error; MLR: multiple linear regression; MSE: mean square error; MTFF-ANN: multitype feature fusion artificial neural network (2 CNN+1 LSTM); PIR: photoplethysmogram intensity ratio; PPG: photoplethysmography; PPT: pulse transit time; RF: random forest; RMSE: root mean square error; RNN: recurrent neural networks; SE: standard error; SSR: state space reconstruction; MARS: multiadaptive regression spline; WkNN: weighted *k*-near neighbor.

## Data Availability

We can send the datasets at the request of the authors. The data was obtained from the IEEE Dataport open source site.
